RETRACTED

# Analysis of Communication and Network Securities Using the Concepts of Complex Picture Fuzzy Relations

**DOI:** 10.1155/2021/9427492

**Published:** 2021-10-31

**Authors:** Abdul Nasir, Naeem Jan, Sami Ullah Khan, Abdu Gumaei, Abdulrahman Alothaim

**Affiliations:** ^1^Department of Mathematics, Institute of Numerical Sciences, Gomal University, Dera Ismail Khan 29050, Khyber Pakhtunkhwa, Pakistan; ^2^Computer Science Department, Faculty of Applied Sciences, Taiz University, Taiz 6803, Yemen; ^3^STC's Artificial Intelligence Chair, Department of Information Systems, College of Computer and Information Sciences, King Saud University, Riyadh 11543, Saudi Arabia

## Abstract

In our lives, we cannot avoid the uncertainty. Randomness, rough knowledge, and vagueness lead us to uncertainty. In mathematics, the fuzzy set (FS) theory and logics are used to model uncertain events. This article defines a new concept of complex picture fuzzy relation (CPFR) in the field of FS theory. In addition, the types of CPFRs are also discussed to make the paper more fruitful. Today's complex network architecture faces the ever-changing threats. The cyber-attackers are always trying to discover, catch, and exploit the weaknesses in the networks. So, the security measures are essential to avoid and dismantle such threats. The CPFR has a vast structure composed of levels of membership, abstinence, and nonmembership which models uncertainty better than any other structures in the theory. Moreover, a CPFR has the ability to cope with multivariable problems. Therefore, this article proposes modeling techniques based on the complex picture fuzzy information which are used to study the effectiveness and ineffectiveness of different network securities against several threats and cyber-attack practices. Moreover, the strength and preeminence of the proposed methods are verified by studying their comparison with the existing methods.

## 1. Introduction

Uncertainty is an inevitable part of human life which has many causes ranging from just falling short of conviction to almost complete absence of awareness or belief. Probability measures the uncertainty due to randomness. Mostly mathematics deals with precise and accurate information. Modeling uncertainty has long been a crux for mathematicians. In 1965, fuzzy sets (FSs) and logics were presented by Zadeh [1] which deal with uncertainty and vagueness or fuzziness. A FS assigns the level of membership to every element in the set. The level of membership is a function that takes on the values from the unit interval [0,  1].

Klir and Folger [2] defined the relations between classical sets. A relation of classical sets (classical relation) specifies the existence and nonexistence of a relationship, i.e., the classical set theory only works with the problems of yes-and-no-type. Mendel [3] introduced the relations for FS, known as fuzzy relations (FRs). Unlike classical relations, FRs are not restricted to yes-or-no type problems. The level of membership enables them to specify the level, strength, and grade of good or healthy relations between any pair of FSs. The higher values of level of membership indicate that the relation is a strong relation, while the lower values are the indication of weak relationship. FR is a broader concept than a classical relation, and it can handle the problems in both the environments. If we assign the values of membership as 0 and 1, then a FR becomes a classical relation. Tamir et al. [4] proposed an overview of theory and applications of CFSs, Nasir et al. [5] carried out the medical diagnosis and life span of ill people using the interval-valued CFRs, Bi et al. [6] studied the parallelism of CFSs, Feng et al. [7] came up with the idea of multiple FRs and their application to coupled fuzzy control, and Al-Quduh and Hassan [8] used uncertain periodic data and applied the CFRs in decision makings.

RETRACTED

Atanassov [9] realized that a FS can become stronger if the level of nonmembership is included to its structure because it was felt that there are many situations where FS cannot be applied due to its limitation. So, he initiated the intuitionistic FS (IFS). According to Atanassov, the values assigned to level of membership and level of nonmembership must be from the unit interval [0, 1], such that the sum of both the values also ends up between 0 and 1. The improvement in the structure of an IFS as compared with the structure of FS is that an IFS talks over the level of satisfaction represented by the level of membership as well as the level of dissatisfaction represented by the level of nonmembership. Burillo and Bustince [10] devised the conception of intuitionistic FR (IFR) which studies the relationships between any IFSs.

Later, Cuong [11] defined the picture FSs (PFSs) by the addition of level of abstinence in the structure of IFS. In a PFS, the level of membership, level of abstinence, and level of nonmembership take on values from the unit interval provided that their sum is between 0 and 1. Szmidt and Kacprzyk [12] found the distance between IFSs, Atanassov [13] defined new operators over IFSs, De et al. [14] carried out some operations on IFSs, and Deschrijver and Kerre [15] wrote on the composition of IFRs. Bustince [16] constructed the IFRs with predetermined properties, Ejegwa [17] improved the composite relation for PyFSs and applied them in medical diagnosis, Mahmood [18] proposed the application of bipolar soft sets, Phong et al. [19] offered some composition of picture FRs (PFRs), Van Dinh et al. [20] presented the theories and applications of picture fuzzy database, Cuong and Kreinovich [21] proposed a new concept of PFSs for the problems in computational intelligence, and Dutta [22] used the PFSs for medical diagnosis.

RETRACTED

Ramot et al. [23] introduced the notion of complex FS (CFS). They switched the range of a level of membership to a complex number in the unit circle in a complex plane. The complex valued membership is expressed in the polar form, i.e., *α*(*d*)*e*^2*ρ*(*d*)*πj*^. The base term *α*(*d*) is called the amplitude term, and the term in exponent *ρ*(*d*) is called the phase term. This complex structure with dual parts enables the CFSs to model the problems with multivariable. Further, the complex FR (CFR) was defined by Ramot et al. [23]. Alkouri and Salleh [24] introduced the complex IFSs (CIFSs) which consist of both the levels of membership and nonmembership provided that the values and their sum are contained in the unit circle in a complex plane. The level of abstinence was missing in the structure of CIFSs, so Akram et al. [25] defined the complex PFSs (CPFSs). The CPFSs assign the level of membership, level of abstinence, and level of nonmembership to each of the set members which range between 0 and 1. The values assigned are such that their sum does not exceed 1. Yazdanbakhsh and Dick [26] reviewed the CFSs, Dick [27] studied the complex fuzzy logic, Nasir et al. [28–31] proposed rich applications of complex fuzzy relations and its generalizations, Thirunavukarasu et al. [32] proposed the applications of CFSs, Ngan et al. [33] applied and represented the CIFS by quaternion numbers, Alkouri and Salleh [34] worked on complex IFRs (CIFRs), and Yaqoob et al. [35] applied the CIFRs to cellular network provide companies. Jan et al. [36, 37] initiated the innovative concepts of CIFRs and IVCIFRs and proposed the applications of said concepts in the analysis of cyber-securities, cyber threats in petroleum sectors, and other industries. Lin et al. [38–40] worked comprehensively on decision-making techniques in the environment of picture fuzzy information. Xu et al. [41] followed an approach based rough FS to detect the frauds in telecommunication, Pithani and Sethi [42] worked on a fuzzy set delay representation for computer network routing algorithms, Fu et al. [43] assessed the information systems security risk on FS, Biswas et al. [44] proposed the intuitionistic fuzzy real time multigraphs for communication networks, and Gao and Feng [45] used rough FS for risk evaluation of the electric power communication network.

RETRACTED

In this article, the complex PFSs (CPFSs) and the innovative concepts of complex picture fuzzy relations (CPFRs) are studied. These structures talk about the level of membership, level of abstinence, and level of nonmembership. The sum of all the three level values must lie within the unit circle in the complex plane. Moreover, the Cartesian product between two CPFSs is introduced. Now, by the introduction of CPFRs, we can find out the relationships between any two CPFSs. Furthermore, the types of CPFSs are discussed through various examples, theorems, and definitions. The types include complex picture reflexive fuzzy relation (CP-reflexive-FR), CP-irreflexive-FR, CP-symmetric-FR, CP-antisymmetric-FR, CP-asymmetric-FR, CP-transitive-FR, CP-composite-FR, CP-equivalence-FR, CP-preorder-FR, CP-partial order-FR, CP-complete-FR, CP-linear order-FR, CP-strict order-FR, converse of a CPFR, and the equivalence classes for CP-equivalence-FR. In addition, the CPFRs have the capacity to deal with the multivariable problems. They have a diverse structure, which can process the information of many types including fuzzy, complex fuzzy, intuitionistic fuzzy, intuitionistic fuzzy, picture fuzzy, and complex picture fuzzy information. These facts clearly define the advantage of the proposed structure over other existing structures.

This article also proposes a novel technique for fuzzy modeling which is based on the proposed concepts of CPFSs and CPFRs. As an illustration, the said modeling technique is applied to solve the network security problems. Network security is an expansive word that covers a group of technologies, devices, techniques, and procedures. Basically, the network security aims to protect and maintain the reliability, privacy, and availability of data and computer networks using software and hardware technologies. In order to obtain those goals, it designs a collection of procedures and alignments. In today's digital world, it has become the fundamental necessity of companies, industries, businesses, and organizations. They need protection from the escalating cyber threats. Observing the significance of the issue, we introduced a modeling technique for an analysis (Figure 1).

The CPFR is a tool that finds out and analyzes the relationship between the CPFSs. This article is aimed to study the effects of different communication network securities and the threats to those networks. For that reason, an efficient structure of CPFS is used because it has the abilities to model uncertainty in all aspects, i.e., positive effects, no effects, and negative effects with respect to some time frame. Therefore, to investigate the relationships among the set of network securities and threats, the CPFRs and their types are used. In addition, this application problem is solved using preexisting frameworks which all fail to model it to the requirements. Further, these methods can be extended to other structures of fuzzy set theory that will produce robust modeling techniques which can be used in economics, statistics, computer sciences, information technology fields, engineering, sports, and medical fields.

RETRACTED

The organization of this article is given in Table 1.

## 2. Preliminaries

In this section, the definitions and examples of fundamental concepts are reviewed, which include FSs, CFSs, IFSs, CIFSs, PFSs, CPFSs, and Cartesian product of two CFSs and CFRs.

**Definition 1 (see [1]).**

Let *Y* be a universe and *D* be a collection of elements in *Y*. Then, *D* is called a fuzzy set (FS) if it is of the form as follows:

(1) $$\begin{array}{c} D=\left\{d,m\left(d\right):\;d\in Y\right\}, \end{array}$$

where *m*(*d*) : *Y*⟶[0,1] symbolizes the level of membership of *D*.

**Definition 2 (see [23]).**

Let *Y* be a universe and *D* be a collection of elements in *Y*. Then, *D* is called a complex fuzzy set (CFS) if

(2) $$\begin{array}{c} D=\left\{d,M\left(d\right):\;d\in Y\right\}, \end{array}$$

where *M*(*d*) : *Y*⟶{*z* :  *z* ∈ *ℂ*, |*z*| ≤ 1} symbolizes the level of membership of *D* and *z* is a complex number. Another form of a CFS is

(3) $$\begin{array}{c} D=\left\{d,\alpha \left(d\right)e^{2\rho \left(d\right)\pi j}:\;d\in Y\right\}, \end{array}$$

where $j=\sqrt{-1}$, *α*(*d*) : *Y*⟶[0,1] is called the amplitude value of level of membership, and *ρ*(d) : *Y*⟶[0,1] is called the phase value of level of membership.

**Definition 3 (see [23]).**

If *D*={*d*, *α*(*d*)*e*^2*ρ*(*d*)*πj*^ :  *d* ∈ *Y*} and *F*={*f*, *α*(*f*)*e*^2*ρ*(*f*)*πj*^ :  *f* ∈ *Y*} are two CFSs in universe *Y*, then the Cartesian product between *D* and *F* is given as follows:

(4) $$\begin{array}{c} D\times F=\left\{\left(d,f\right),\alpha \left(d,f\right)e^{2\rho \left(d,f\right)\pi j}:d\in D,f\in F\right\}, \end{array}$$

where *α*(*d*, *f*) : *Y*⟶[0,1] and *ρ*(*d*, *f*) : *Y*⟶[0,1] symbolize the amplitude value and phase value of the level of membership of the Cartesian product *D* × *F* defined as follows:

(5) $$\begin{array}{c} \alpha \left(d,f\right)=\min\left\{\alpha \left(d\right),\alpha \left(f\right)\right\},\\ \rho \left(d,f\right)=\min\left\{\rho \left(d\right),\rho \left(f\right)\right\}. \end{array}$$

**Definition 4 (see [23]).**

Any subcollection of a Cartesian product between two CFSs is said to be a complex fuzzy relation (CFR) which is denoted by *R*, i.e., *R*⊆*D* × *F*.

RETRACTED

**Example 1 .**

If *D*={(*d*, (2/3)*e*^2(1/2)*πj*^), (*f*, (2/5)*e*^2(2/3)*πj*^), (*g*, (2/7)*e*^2(3/5)*πj*^)} is a CFS, then the Cartesian product on *D* is

(6) $$\begin{array}{c} D\times D=\left\{\begin{array}{c} \left(\left(d,d\right),\frac{2}{3}e^{2\left(1/2\right)\pi j}\right),\left(\left(d,f\right),\frac{2}{5}e^{2\left(1/2\right)\pi j}\right),\left(\left(d,g\right),\frac{2}{7}e^{2\left(1/2\right)\pi j}\right),\\ \left(\left(f,d\right),\frac{2}{5}e^{2\left(1/2\right)\pi j}\right),\left(\left(f,f\right),\frac{2}{5}e^{2\left(2/3\right)\pi j}\right),\left(\left(f,g\right),\frac{2}{7}e^{2\left(3/5\right)\pi j}\right),\\ \left(\left(g,d\right),\frac{2}{7}e^{2\left(1/2\right)\pi j}\right),\left(\left(g,f\right),\frac{2}{7}e^{2\left(3/5\right)\pi j}\right),\left(\left(g,g\right),\frac{2}{7}e^{2\left(3/5\right)\pi j}\right). \end{array}\right\} \end{array}$$

The CFR *R* is

(7) $$\begin{array}{c} R=\left\{\begin{array}{c} \left(\left(d,d\right),\frac{2}{3}e^{2\left(1/2\right)\pi j}\right),\left(\left(d,f\right),\frac{2}{5}e^{2\left(1/2\right)\pi j}\right),\left(\left(f,g\right),\frac{2}{7}e^{2\left(3/5\right)\pi j}\right),\\ \left(\left(g,f\right),\frac{2}{7}e^{2\left(3/5\right)\pi j}\right),\left(\left(g,g\right),\frac{2}{7}e^{2\left(3/5\right)\pi j}\right). \end{array}\right\} \end{array}$$

**Definition 5 (see [9]).**

Let *Y* be a universe and *D* be a collection of elements in *Y*. Then, *D* is called an intuitionistic fuzzy set (IFS) if it is of the form as follows:

(8) $$\begin{array}{c} D=\left\{d,m\left(d\right),n\left(d\right):\;d\in Y\right\}, \end{array}$$

where *m*(*d*) : *Y*⟶[0,1] symbolizes the level of membership of *D* and *n*(*d*) : *Y*⟶[0,1] symbolizes the level of nonmembership of *D* such that 0 ≤ *m*(*d*)+*n*(*d*) ≤ 1.

**Definition 6 (see [24]).**

Let *Y* be a universe and *D* be a collection of elements in *Y*. Then, *D* is called a complex intuitionistic fuzzy set (CIFS) if

(9) $$\begin{array}{c} D=\left\{d,M\left(d\right),N\left(d\right):\;d\in Y\right\}, \end{array}$$

where *M*(*d*) : *Y*⟶{*z*_1_ :  *z*_1_ ∈ *ℂ*, |*z*_1_| ≤ 1} symbolizes the level of membership of *D*, *N*(*d*) : *Y*⟶{*z*_2_ :  *z*_2_ ∈ *ℂ*, |*z*_2_| ≤ 1} symbolizes the level of nonmembership of *D*, and *z*_1_ and *z*_2_ are complex numbers such that 0 ≤ |*z*_1_|+|*z*_2_| ≤ 1. Another form of a CIFS is

(10) $$\begin{array}{c} D=\left\{d,\alpha_{M}\left(d\right)e^{2\rho_{M}\left(d\right)\pi j},\alpha_{N}\left(d\right)e^{2\rho_{N}\left(d\right)\pi j}:\;d\in Y\right\}, \end{array}$$

where $j=\sqrt{-1}$, *α*_*M*_(*d*) : *Y*⟶[0,1] is called the amplitude value of level of membership, *ρ*_*M*_(d) : *Y*⟶[0,1] is called the phase value of level of membership, *α*_*N*_(*d*) : *Y*⟶[0,1] is called the amplitude value of level of nonmembership, and *ρ*_*N*_(*d*) : *Y*⟶[0,1] is called the phase value of level of nonmembership such that 0 ≤ *α*_*M*_(*d*)+*α*_*N*_(*d*) ≤ 1 and 0 ≤ *ρ*_*M*_(*d*)+*ρ*_*N*_(*d*) ≤ 1.

RETRACTED

**Definition 7 (see [11]).**

Let *Y* be a universe and *D* be a collection of elements in *Y*. Then, *D* is called a picture fuzzy set (PFS) if it is of the form

(11) $$\begin{array}{c} D=\left\{d,m\left(d\right),a\left(d\right),\;n\left(d\right):\;d\in Y\right\}, \end{array}$$

where *m*(*d*) : *Y*⟶[0,1] symbolizes the level of membership of *D*, *a*(*d*) : *Y*⟶[0,1] symbolizes the level of abstinence of *D*, and *n*(*d*) : *Y*⟶[0,1] symbolizes the level of nonmembership of *D* such that 0 ≤ *m*(*d*)+*a*(*d*)+*n*(*d*) ≤ 1.

**Definition 8 (see [25]).**

Let *Y* be a universe and *D* be a collection of elements in *Y*. Then, *D* is called a complex picture fuzzy set (CPFS) if

(12) $$\begin{array}{c} D=\left\{d,M\left(d\right),A\left(d\right),N\left(d\right):\;d\in Y\right\}, \end{array}$$

where *M*(*d*) : *Y*⟶{*z*_1_ :  *z*_1_ ∈ *ℂ*, |*z*_1_| ≤ 1} symbolizes the level of membership of *D*, *A*(*d*) : *Y*⟶{*z*_2_ : *z*_2_ ∈ *ℂ*, |*z*_2_| ≤ 1} symbolizes the level of abstinence of *D*, *N*(*d*) : *Y*⟶{*z*_3_ :  *z*_3_ ∈ *ℂ*, |*z*_3_| ≤ 1} symbolizes the level of nonmembership of *D*, and *z*_1_, *z*_2_,  and *z*_3_ are complex numbers such that for any nonnegative integer *q*, 0 ≤ |*z*_1_|+|*z*_2_|+|*z*_3_| ≤ 1. Another form of a CPFS is

(13) $$\begin{array}{c} D=\left\{d,\alpha_{M}\left(d\right)e^{2\rho_{M}\left(d\right)\pi j},\alpha_{A}\left(d\right)e^{2\rho_{A}\left(d\right)\pi j},\;\alpha_{N}\left(d\right)e^{2\rho_{N}\left(d\right)\pi j}:\;d\in Y\right\}, \end{array}$$

where $j=\sqrt{-1}$, *α*_*M*_(*d*) : *Y*⟶[0,1] is called the amplitude value of level of membership, *ρ*_*M*_(*d*) : *Y*⟶[0,1] is called the phase value of level of membership, *α*_*A*_(*d*) : *Y*⟶[0,1] is called the amplitude value of level of abstinence, *ρ*_*A*_(*d*) : *Y*⟶[0,1] is called the phase value of level of abstinence, *α*_*N*_(*d*) : *Y*⟶[0,1] is called the amplitude value of level of nonmembership, and *ρ*_*N*_(*d*) : *Y*⟶[0,1] is called the phase value of level of nonmembership such that 0 ≤ *α*_*M*_(*d*)+*α*_*A*_(*d*)+*α*_*N*_(*d*) ≤ 1 and 0 ≤ *ρ*_*M*_(*d*)+*ρ*_*A*_(*d*)+*ρ*_*N*_(*d*) ≤ 1.

## 3. Complex Picture Fuzzy Relations

In this section, the novel concepts of complex picture fuzzy relation (CPFR), Cartesian products between two CPFSs, and different types of CPFRs are introduced. Every definition is supported by an example.

**Definition 9 .**

If *D*={*d*, *α*_*M*_(*d*)*e*^2*ρ*_*M*_(*d*)*πj*^, *α*_*A*_(*d*)*e*^2*ρ*_*A*_(*d*)*πj*^,  *α*_*N*_(*d*)*e*^2*ρ*_*N*_(*d*)*πj*^ :  *d* ∈ *Y*} and *F*={*d*, *α*_*M*_(*f*)*e*^2*ρ*_*M*_(*f*)*πj*^, *α*_*A*_(*f*)*e*^2*ρ*_*A*_(*f*)*πj*^,  *α*_*N*_(*f*)*e*^2*ρ*_*N*_(*f*)*πj*^ :  *d* ∈ *Y*} are two CPFSs in universe *Y*, then the Cartesian product between *D* and *F* is given as follows:

(14) $$\begin{array}{c} D\times F=\left\{\left(d,f\right),\alpha_{M}\left(d,f\right)e^{2\rho_{M}\left(d,f\right)\pi j},\alpha_{A}\left(d,f\right)e^{2\rho_{A}\left(d,f\right)\pi j},\;\alpha_{N}\left(d,f\right)e^{2\rho_{N}\left(d,f\right)\pi j}:\;d\in D,f\in F\right\}, \end{array}$$

where *α*_*M*_(*d*, *f*) : *Y*⟶[0,1], *α*_*N*_(*d*, *f*) : *Y*⟶[0,1], and  *α*_*N*_(*d*, *f*) : *Y*⟶[0,1] symbolize the amplitude values of levels of membership, abstinence, and nonmembership of the Cartesian product *D* × *F*, respectively. *ρ*_*M*_(*d*, *f*) : *Y*⟶[0,1], *ρ*_*N*_(*d*, *f*) : *Y*⟶[0,1], and  *ρ*_*N*_(*d*, *f*) : *Y*⟶[0,1] symbolize the phase values of levels of membership, abstinence, and nonmembership of the Cartesian product *D* × *F*, respectively. These values for *D* × *F* are defined as

(15) $$\begin{array}{c} \alpha_{M}\left(d,f\right)=\min\left\{\alpha_{M}\left(d\right),\alpha_{M}\left(f\right)\right\},\\ \rho_{M}\left(d,f\right)=\min\left\{\rho_{M}\left(d\right),\rho_{M}\left(f\right)\right\},\\ \alpha_{A}\left(d,f\right)=\min\left\{\alpha_{A}\left(d\right),\alpha_{A}\left(f\right)\right\},\\ \rho_{A}\left(d,f\right)=\min\left\{\rho_{A}\left(d\right),\rho_{A}\left(f\right)\right\},\\ \alpha_{N}\left(d,f\right)=\max\left\{\alpha_{N}\left(d\right),\alpha_{N}\left(f\right)\right\},\\ \rho_{N}\left(d,f\right)=\max\left\{\rho_{N}\left(d\right),\rho_{N}\left(f\right)\right\}. \end{array}$$

**Definition 10 .**

RETRACTED

Any subcollection of a Cartesian product of two CPFSs is said to be a complex fuzzy relation (CPFR) which is denoted by *R*, i.e., *R*⊆*D* × *F*.

**Example 2 .**

If

(16) $$\begin{array}{c} D=\left\{\begin{array}{c} \left(d,\frac{1}{3}e^{2\left(1/20\right)\pi j},\frac{1}{5}e^{2\left(1/10\right)\pi j},\frac{1}{3}e^{2\left(1/4\right)\pi j}\right),\left(f,\frac{2}{5}e^{2\left(1/5\right)\pi j},\frac{2}{5}e^{2\left(3/10\right)\pi j},\frac{1}{5}e^{2\left(1/5\right)\pi j}\right),\\ \left(g,\frac{2}{7}e^{2\left(1/10\right)\pi j},\frac{3}{10}e^{2\left(7/10\right)\pi j},\frac{1}{4}e^{2\left(1/6\right)\pi j}\right), \end{array}\right\} \end{array}$$

is a CPFS, then the Cartesian product is *D* × *D*{((*d*, *d*), 1/3*e*^2(1/20)*πj*^, 1/5*e*^2(1/10)*πj*^, 1/3*e*^2(1/4)*πj*^), ((*d*, *f*), 1/3*e*^2(1/20)*πj*^, 1/5*e*^2(1/10)*πj*^, 1/3*e*^2(1/4)*πj*^), ((*d*, *g*), 2/7*e*^2(1/20)*πj*^, 1/5*e*^2(1/10)*πj*^, 1/3*e*^2(1/4)*πj*^), ((*f*, *d*), 1/3*e*^2(1/20)*πj*^, 1/5*e*^2(1/10)*πj*^, 1/3*e*^2(1/4)*πj*^), ((*f*, *f*), 2/5*e*^2(1/5)*πj*^, 2/5*e*^2(3/10)*πj*^, 2/10*e*^2(1/5)*πj*^), ((*f*, *g*), 2/7*e*^2(1/10)*πj*^, 3/10*e*^2(3/10)*πj*^, 1/4*e*^2(1/5)*πj*^), ((*g*, *d*), 2/7*e*^2(1/10)*πj*^, 1/5*e*^2(1/10)*πj*^, 1/3*e*^2(1/4)*πj*^), ((*g*, *h*), 2/7*e*^2(1/10)*πj*^, 3/10*e*^2(3/10)*πj*^, 1/4*e*^2(1/5)*πj*^), ((*g*, *g*), 2/7*e*^2(1/10)*πj*^, 3/10*e*^2(7/10)*πj*^, 1/4*e*^2(1/6)*πj*^)}

The CPFR *R* is

(17) $$\begin{array}{c} R=\left\{\begin{array}{c} \left(\left(d,d\right),\frac{1}{3}e^{2\left(1/20\right)\pi j},\frac{1}{5}e^{2\left(1/10\right)\pi j},\frac{1}{3}e^{2\left(1/4\right)\pi j}\right),\left(\left(f,d\right),\frac{1}{3}e^{2\left(1/20\right)\pi j},\frac{1}{5}e^{2\left(1/10\right)\pi j},\frac{1}{3}e^{2\left(1/4\right)\pi j}\right),\\ \left(\left(g,f\right),\frac{2}{7}e^{2\left(1/10\right)\pi j},\frac{3}{10}e^{2\left(3/10\right)\pi j},\frac{1}{4}e^{2\left(1/5\right)\pi j}\right),\left(\left(g,g\right),\frac{2}{7}e^{2\left(1/10\right)\pi j},\frac{3}{10}e^{2\left(7/10\right)\pi j},\frac{1}{4}e^{2\left(1/6\right)\pi j}\right). \end{array}\right\} \end{array}$$

**Definition 11 .**

RETRACTED

The converse of a CPFR

*R*={(*d*, *f*), *α*_*M*_(*d*, *f*)*e*^2*ρ*_*M*_(*d*, *f*)*πj*^, *α*_*A*_(*d*, *f*)*e*^2*ρ*_*A*_(*d*, *f*)*πj*^,  *α*_*N*_(*d*, *f*)*e*^2*ρ*_*N*_(*d*, *f*)*πj*^ :  (*d*, *f*) ∈ *R*} is defined as *R*^−1^={(*f*, *d*), *α*_*M*_(*f*, *d*)*e*^2*ρ*_*M*_(*f*, *d*)*πj*^, *α*_*A*_(*f*, *d*)*e*^2*ρ*_*A*_(*f*, *d*)*πj*^,  *α*_*N*_(*f*, *d*)*e*^2*ρ*_*N*_(*f*, *d*)*πj*^ :  (*d*, *f*) ∈ *R*}.

**Example 3 .**

The converse of CPFR *R* given as follows:

(18) $$\begin{array}{c} R=\left\{\begin{array}{c} \left(\left(d,d\right),\frac{1}{3}e^{2\left(1/20\right)\pi j},\frac{1}{5}e^{2\left(1/10\right)\pi j},\frac{1}{3}e^{2\left(1/4\right)\pi j}\right),\left(\left(f,d\right),\frac{1}{3}e^{2\left(1/20\right)\pi j},\frac{1}{5}e^{2\left(1/10\right)\pi j},\frac{1}{3}e^{2\left(1/4\right)\pi j}\right)\\ \left(\left(g,f\right),\frac{2}{7}e^{2\left(1/10\right)\pi j},\frac{3}{10}e^{2\left(3/10\right)\pi j},\frac{1}{4}e^{2\left(1/5\right)\pi j}\right),\left(\left(g,g\right),\frac{2}{7}e^{2\left(1/10\right)\pi j},\frac{3}{10}e^{2\left(7/10\right)\pi j},\frac{1}{4}e^{2\left(1/6\right)\pi j}\right) \end{array}\right\}, \end{array}$$

is

(19) $$\begin{array}{c} R^{-1}=\left\{\begin{array}{c} \left(\left(d,d\right),\frac{1}{3}e^{2\left(1/20\right)\pi j},\frac{1}{5}e^{2\left(1/10\right)\pi j},\frac{1}{3}e^{2\left(1/4\right)\pi j}\right),\left(\left(d,f\right),\frac{1}{3}e^{2\left(1/20\right)\pi j},\frac{1}{5}e^{2\left(1/10\right)\pi j},\frac{1}{3}e^{2\left(1/4\right)\pi j}\right)\\ \left(\left(f,g\right),\frac{2}{7}e^{2\left(1/10\right)\pi j},\frac{3}{10}e^{2\left(3/10\right)\pi j},\frac{1}{4}e^{2\left(1/5\right)\pi j}\right),\left(\left(g,g\right),\frac{2}{7}e^{2\left(1/10\right)\pi j},\frac{3}{10}e^{2\left(7/10\right)\pi j},\frac{1}{4}e^{2\left(1/6\right)\pi j}\right) \end{array}\right\}. \end{array}$$

**Definition 12 .**

RETRACTED

A CPFR *R* is a complex picture reflexive fuzzy relation (CP-reflexive-FR) if ∀(*d*, *α*_*M*_(*d*)*e*^2*ρ*_*M*_(*d*)*πj*^, *α*_*A*_(*d*)*e*^2*ρ*_*A*_(*d*)*πj*^,  *α*_*N*_(*d*)*e*^2*ρ*_*N*_(*d*)*πj*^) ∈ *D* implies ((*d*, *d*), *α*_*M*_(*d*, *d*)*e*^2*ρ*_*M*_(*d*, *d*)*πj*^, *α*_*A*_(*d*, *d*)*e*^2*ρ*_*A*_(*d*, *d*)*πj*^,  *α*_*N*_(*d*, *d*)*e*^2*ρ*_*N*_(*d*, *d*)*πj*^) ∈ *R*.

**Example 4 .**

The relation *R* is a CP-reflexive-FR on a CPFS *D* as follows:

(20) $$\begin{array}{c} D=\left\{\begin{array}{c} \left(d,\frac{1}{3}e^{2\left(1/20\right)\pi j}.\frac{1}{5}e^{2\left(1/10\right)\pi j},\frac{1}{3}e^{2\left(1/4\right)\pi j}\right),\left(f,\frac{2}{5}e^{2\left(1/5\right)\pi j},\frac{2}{5}e^{2\left(3/10\right)\pi j},\frac{1}{5}e^{2\left(1/5\right)\pi j}\right)\\ \left(g,\frac{2}{7}e^{2\left(1/10\right)\pi j},\frac{3}{10}e^{2\left(7/10\right)\pi j},\frac{1}{4}e^{2\left(1/6\right)\pi j}\right) \end{array}\right\},\\ R=\left\{\begin{array}{c} \left(\left(d,d\right),\frac{1}{3}e^{2\left(1/20\right)\pi j},\frac{1}{5}e^{2\left(1/10\right)\pi j},\frac{1}{3}e^{2\left(1/4\right)\pi j}\right),\left(\left(f,f\right),\frac{2}{5}e^{2\left(1/5\right)\pi j},\frac{2}{5}e^{2\left(3/10\right)\pi j},\frac{2}{10}e^{2\left(1/5\right)\pi j}\right)\\ \left(\left(g,g\right),\frac{2}{7}e^{2\left(1/10\right)\pi j},\frac{3}{10}e^{2\left(7/10\right)\pi j},\frac{1}{4}e^{2\left(1/6\right)\pi j}\right) \end{array}\right\}. \end{array}$$

**Definition 13 .**

A CPFR *R* is a complex picture irreflexive fuzzy relation (CP-irreflexive-FR) if ∀(*d*, *α*_*M*_(*d*)*e*^2*ρ*_*M*_(*d*)*πj*^, *α*_*A*_(*d*)*e*^2*ρ*_*A*_(*d*)*πj*^,  *α*_*N*_(*d*)*e*^2*ρ*_*N*_(*d*)*πj*^) ∈ *D* implies ((*d*, *d*), *α*_*M*_(*d*, *d*)*e*^2*ρ*_*M*_(*d*, *d*)*πj*^, *α*_*A*_(*d*, *d*)*e*^2*ρ*_*A*_(*d*, *d*)*πj*^,  *α*_*N*_(*d*, *d*)*e*^2*ρ*_*N*_(*d*, *d*)*πj*^) ∉ *R*.

**Example 5 .**

The following relation *R* is a CP-irreflexive-FR on a CPFS *D* given in equation (20):

(21) $$\begin{array}{c} R=\left\{\begin{array}{c} \left(\left(d,f\right),\frac{1}{3}e^{2\left(1/20\right)\pi j},\frac{1}{5}e^{2\left(1/10\right)\pi j},\frac{1}{3}e^{2\left(1/4\right)\pi j}\right),\left(\left(d,g\right),\frac{2}{7}e^{2\left(1/20\right)\pi j},\frac{1}{5}e^{2\left(1/10\right)\pi j},\frac{1}{3}e^{2\left(1/4\right)\pi j}\right)\\ \left(\left(f,d\right),\frac{1}{3}e^{2\left(1/20\right)\pi j},\frac{1}{5}e^{2\left(1/10\right)\pi j},\frac{1}{3}e^{2\left(1/4\right)\pi j}\right),\left(\left(f,g\right),\frac{2}{7}e^{2\left(1/10\right)\pi j},\frac{3}{10}e^{2\left(3/10\right)\pi j},\frac{1}{4}e^{2\left(1/5\right)\pi j}\right)\\ \left(\left(g,d\right),\frac{2}{7}e^{2\left(1/20\right)\pi j},\frac{1}{5}e^{2\left(1/10\right)\pi j},\frac{1}{3}e^{2\left(1/4\right)\pi j}\right) \end{array}\right\}. \end{array}$$

**Definition 14 .**

RETRACTED

A CPFR *R* is a complex picture symmetric fuzzy relation (CP-symmetric-FR) if ((*d*, *f*), *α*_*M*_(*d*, *f*)*e*^2*ρ*_*M*_(*d*, *f*)*πj*^, *α*_*A*_(*d*, *f*)*e*^2*ρ*_*A*_(*d*, *f*)*πj*^,  *α*_*N*_(*d*, *f*)*e*^2*ρ*_*N*_(*d*, *f*)*πj*^) ∈ *R* implies ((*f*, *d*), *α*_*M*_(*f*, *d*)*e*^2*ρ*_*M*_(*f*, *d*)*πj*^, *α*_*A*_(*f*, *d*)*e*^2*ρ*_*A*_(*f*, *d*)*πj*^,  *α*_*N*_(*f*, *d*)*e*^2*ρ*_*N*_(*f*, *d*)*πj*^) ∈ *R*.

**Example 6 .**

The following relation *R* is a CP-symmetric-FR on a CPFS *D* given in equation (20):

(22) $$\begin{array}{c} R=\left\{\begin{array}{c} \left(\left(d,d\right),\frac{1}{3}e^{2\left(1/20\right)\pi j},\frac{1}{5}e^{2\left(1/10\right)\pi j},\frac{1}{3}e^{2\left(1/4\right)\pi j}\right),\left(\left(d,f\right),\frac{1}{3}e^{2\left(1/20\right)\pi j},\frac{1}{5}e^{2\left(1/10\right)\pi j},\frac{1}{3}e^{2\left(1/4\right)\pi j}\right)\\ \left(\left(f,d\right),\frac{1}{3}e^{2\left(1/20\right)\pi j},\frac{1}{5}e^{2\left(1/10\right)\pi j},\frac{1}{3}e^{2\left(1/4\right)\pi j}\right),\left(\left(f,f\right),\frac{2}{5}e^{2\left(1/5\right)\pi j},\frac{2}{5}e^{2\left(3/10\right)\pi j},\frac{2}{10}e^{2\left(1/5\right)\pi j}\right)\\ \left(\left(f,g\right),\frac{2}{7}e^{2\left(1/10\right)\pi j},\frac{3}{10}e^{2\left(3/10\right)\pi j},\frac{1}{4}e^{2\left(1/5\right)\pi j}\right),\left(\left(g,f\right),\frac{2}{7}e^{2\left(1/10\right)\pi j},\frac{3}{10}e^{2\left(3/10\right)\pi j},\frac{1}{4}e^{2\left(1/5\right)\pi j}\right) \end{array}\right\}. \end{array}$$

**Definition 15 .**

A CPFR *R* is a complex picture asymmetric fuzzy relation (CP-asymmetric-FR) if ((*d*, *f*), *α*_*M*_(*d*, *f*)*e*^2*ρ*_*M*_(*d*, *f*)*πj*^, *α*_*A*_(*d*, *f*)*e*^2*ρ*_*A*_(*d*, *f*)*πj*^,  *α*_*N*_(*d*, *f*)*e*^2*ρ*_*N*_(*d*, *f*)*πj*^) ∈ *R* implies ((*f*, *d*), *α*_*M*_(*f*, *d*)*e*^2*ρ*_*M*_(*f*, *d*)*πj*^, *α*_*A*_(*f*, *d*)*e*^2*ρ*_*A*_(*f*, *d*)*πj*^,  *α*_*N*_(*f*, *d*)*e*^2*ρ*_*N*_(*f*, *d*)*πj*^) ∉ *R*.

**Example 7 .**

The following relation *R* is a CP-asymmetric-FR on a CPFS *D* given in equation (20):

(23) $$\begin{array}{c} R=\left\{\begin{array}{c} \left(\left(d,f\right),\frac{1}{3}e^{2\left(1/20\right)\pi j},\frac{1}{5}e^{2\left(1/10\right)\pi j},\frac{1}{3}e^{2\left(1/4\right)\pi j}\right),\left(\left(d,g\right),\frac{2}{7}e^{2\left(1/20\right)\pi j},\frac{1}{5}e^{2\left(1/10\right)\pi j},\frac{1}{3}e^{2\left(1/4\right)\pi j}\right)\\ \left(\left(g,f\right),\frac{2}{7}e^{2\left(1/10\right)\pi j},\frac{3}{10}e^{2\left(3/10\right)\pi j},\frac{1}{4}e^{2\left(1/5\right)\pi j}\right) \end{array}\right\}. \end{array}$$

**Definition 16 .**

RETRACTED

A CPFR *R* is a complex picture antisymmetric fuzzy relation (CP-antisymmetric-FR) if ((*d*, *f*), *α*_*M*_(*d*, *f*)*e*^2*ρ*_*M*_(*d*, *f*)*πj*^, *α*_*A*_(*d*, *f*)*e*^2*ρ*_*A*_(*d*, *f*)*πj*^,  *α*_*N*_(*d*, *f*)*e*^2*ρ*_*N*_(*d*, *f*)*πj*^) ∈ *R* and ((*f*, *d*), *α*_*M*_(*f*, *d*)*e*^2*ρ*_*M*_(*f*, *d*)*πj*^, *α*_*A*_(*f*, *d*)*e*^2*ρ*_*A*_(*f*, *d*)*πj*^,  *α*_*N*_(*f*, *d*)*e*^2*ρ*_*N*_(*f*, *d*)*πj*^) ∈ *R* imply

(24) $$\begin{array}{c} \left(\left(d,f\right),\alpha_{M}\left(d,f\right)e^{2\rho_{M}\left(d,f\right)\pi j},\alpha_{A}\left(d,f\right)e^{2\rho_{A}\left(d,f\right)\pi j},\;\alpha_{N}\left(d,f\right)e^{2\rho_{N}\left(d,f\right)\pi j}\right)=\left(\left(f,d\right),\alpha_{M}\left(f,d\right)e^{2\rho_{M}\left(f,d\right)\pi j},\alpha_{A}\left(f,d\right)e^{2\rho_{A}\left(f,d\right)\pi j},\;\alpha_{N}\left(f,d\right)e^{2\rho_{N}\left(f,d\right)\pi j}\right). \end{array}$$

**Example 8 .**

The following relation *R* is a CP-antisymmetric-FR on a CPFS *D* given in equation (20):

(25) $$\begin{array}{c} R=\left\{\begin{array}{c} \left(\left(d,d\right),\frac{1}{3}e^{2\left(1/20\right)\pi j},\frac{1}{5}e^{2\left(1/10\right)\pi j},\frac{1}{3}e^{2\left(1/4\right)\pi j}\right),\left(\left(d,f\right),\frac{1}{3}e^{2\left(1/20\right)\pi j},\frac{1}{5}e^{2\left(1/10\right)\pi j},\frac{1}{3}e^{2\left(1/4\right)\pi j}\right)\\ \left(\left(f,f\right),\frac{2}{5}e^{2\left(1/5\right)\pi j},\frac{2}{5}e^{2\left(3/10\right)\pi j},\frac{2}{10}e^{2\left(1/5\right)\pi j}\right),\left(\left(g,f\right),\frac{2}{7}e^{2\left(1/10\right)\pi j},\frac{3}{10}e^{2\left(3/10\right)\pi j},\frac{1}{4}e^{2\left(1/5\right)\pi j}\right) \end{array}\right\}. \end{array}$$

**Definition 17 .**

A CPFR *R* is a complex picture transitive fuzzy relation (CP-transitive-FR) if ((*d*, *f*), *α*_*M*_(*d*, *f*)*e*^2*ρ*_*M*_(*d*, *f*)*πj*^, *α*_*A*_(*d*, *f*)*e*^2*ρ*_*A*_(*d*, *f*)*πj*^,  *α*_*N*_(*d*, *f*)*e*^2*ρ*_*N*_(*d*, *f*)*πj*^) ∈ *R* and ((*f*, *g*), *α*_*M*_(*f*, *g*)*e*^2*ρ*_*M*_(*f*, *g*)*πj*^, *α*_*A*_(*f*, *g*)*e*^2*ρ*_*A*_(*f*, *g*)*πj*^,  *α*_*N*_(*f*, *g*)*e*^2*ρ*_*N*_(*f*, *g*)*πj*^) ∈ *R* imply ((*d*, *g*), *α*_*M*_(*d*, *g*)*e*^2*ρ*_*M*_(*d*, *g*)*πj*^, *α*_*A*_(*d*, *g*)*e*^2*ρ*_*A*_(*d*, *g*)*πj*^,  *α*_*N*_(*d*, *g*)*e*^2*ρ*_*N*_(*d*, *g*)*πj*^) ∈ *R*.

**Example 9 .**

The following relation *R* is a CP-transitive-FR on a CPFS *D* given in equation (20):

(26) $$\begin{array}{c} R=\left\{\begin{array}{c} \left(\left(d,d\right),\frac{1}{3}e^{2\left(1/20\right)\pi j},\frac{1}{5}e^{2\left(1/10\right)\pi j},\frac{1}{3}e^{2\left(1/4\right)\pi j}\right),\left(\left(d,f\right),\frac{1}{3}e^{2\left(1/20\right)\pi j},\frac{1}{5}e^{2\left(1/10\right)\pi j},\frac{1}{3}e^{2\left(1/4\right)\pi j}\right)\\ \left(\left(d,g\right),\frac{2}{7}e^{2\left(1/20\right)\pi j},\frac{1}{5}e^{2\left(1/10\right)\pi j},\frac{1}{3}e^{2\left(1/4\right)\pi j}\right),\left(\left(f,f\right),\frac{2}{5}e^{2\left(1/5\right)\pi j},\frac{2}{5}e^{2\left(\frac{3}{10}\right)\pi j},\frac{2}{10}e^{2\left(1/5\right)\pi j}\right)\\ \left(\left(g,f\right),\frac{2}{7}e^{2\left(1/10\right)\pi j},\frac{3}{10}e^{2\left(3/10\right)\pi j},\frac{1}{4}e^{2\left(1/5\right)\pi j}\right) \end{array}\right\}. \end{array}$$

**Definition 18 .**

RETRACTED

A CPFR *R* is a complex picture complete fuzzy relation (CP-complete-FR) if ∀(*d*, *α*_*M*_(*d*)*e*^2*ρ*_*M*_(*d*)*πj*^, *α*_*A*_(*d*)*e*^2*ρ*_*A*_(*d*)*πj*^,  *α*_*N*_(*d*)*e*^2*ρ*_*N*_(*d*)*πj*^) ∈ *D* and (*f*, *α*_*M*_(*f*)*e*^2*ρ*_*M*_(*f*)*πj*^, *α*_*A*_(*f*)*e*^2*ρ*_*A*_(*f*)*πj*^,  *α*_*N*_(*f*)*e*^2*ρ*_*N*_(*f*)*πj*^) ∈ *D* imply ((*d*, *f*), *α*_*M*_(*d*, *f*)*e*^2*ρ*_*M*_(*d*, *f*)*πj*^, *α*_*A*_(*d*, *f*)*e*^2*ρ*_*A*_(*d*, *f*)*πj*^,  *α*_*N*_(*d*, *f*)*e*^2*ρ*_*N*_(*d*, *f*)*πj*^) ∈ *R* or ((*f*, *d*), *α*_*M*_(*f*, *d*)*e*^2*ρ*_*M*_(*f*, *d*)*πj*^, *α*_*A*_(*f*, *d*)*e*^2*ρ*_*A*_(*f*, *d*)*πj*^,  *α*_*N*_(*f*, *d*)*e*^2*ρ*_*N*_(*f*, *d*)*πj*^) ∈ *R*.

**Example 10 .**

The following relation *R* is a CP-complete-FR on a CPFS *D* given in equation (20):

(27) $$\begin{array}{c} R=\left\{\begin{array}{c} \left(\left(d,f\right),\frac{1}{3}e^{2\left(1/20\right)\pi j},\frac{1}{5}e^{2\left(1/10\right)\pi j},\frac{1}{3}e^{2\left(1/4\right)\pi j}\right),\left(\left(d,g\right),\frac{2}{7}e^{2\left(1/20\right)\pi j},\frac{1}{5}e^{2\left(1/10\right)\pi j},\frac{1}{3}e^{2\left(1/4\right)\pi j}\right)\\ \left(\left(f,g\right),\frac{2}{7}e^{2\left(1/10\right)\pi j},\frac{3}{10}e^{2\left(3/10\right)\pi j},\frac{1}{4}e^{2\left(1/5\right)\pi j}\right),\left(\left(g,d\right),\frac{2}{7}e^{2\left(1/20\right)\pi j},\frac{1}{5}e^{2\left(1/10\right)\pi j},\frac{1}{3}e^{2\left(1/4\right)\pi j}\right) \end{array}\right\}. \end{array}$$

**Definition 19 .**

A CPFR *R* is a complex picture equivalence fuzzy relation (CP-equivalence-FR) if *R* is

- CP-reflexive-FR
- CP-symmetric-FR
- CP-transitive-FR

**Example 11 .**

The following relation *R* is a CP-equivalence-FR on a CPFS *D* given in equation (20):

(28) $$\begin{array}{c} R=\left\{\begin{array}{c} \left(\left(d,d\right),\frac{1}{3}e^{2\left(1/20\right)\pi j},\frac{1}{5}e^{2\left(1/10\right)\pi j},\frac{1}{3}e^{2\left(1/4\right)\pi j}\right),\left(\left(d,f\right),\frac{1}{3}e^{2\left(1/20\right)\pi j},\frac{1}{5}e^{2\left(1/10\right)\pi j},\frac{1}{3}e^{2\left(1/4\right)\pi j}\right)\\ \left(\left(f,d\right),\frac{1}{3}e^{2\left(1/20\right)\pi j},\frac{1}{5}e^{2\left(1/10\right)\pi j},\frac{1}{3}e^{2\left(1/4\right)\pi j}\right),\left(\left(f,f\right),\frac{2}{5}e^{2\left(1/5\right)\pi j},\frac{2}{5}e^{2\left(\frac{3}{10}\right)\pi j},\frac{2}{10}e^{2\left(1/5\right)\pi j}\right)\\ \left(\left(g,g\right),\frac{2}{7}e^{2\left(1/10\right)\pi j},\frac{3}{10}e^{2\left(7/10\right)\pi j},\frac{1}{4}e^{2\left(1/6\right)\pi j}\right) \end{array}\right\}. \end{array}$$

**Definition 20 .**

RETRACTED

A CPFR *R* is a complex picture preorder fuzzy relation (CP-preorder-FR) if *R* is

- CP-reflexive-FR
- CP-transitive-FR

**Example 12 .**

The following relation *R* is a CP-preorder-FR on a CPFS *D* given in equation (20):

(29) $$\begin{array}{c} R=\left\{\begin{array}{c} \left(\left(d,d\right),\frac{1}{3}e^{2\left(1/20\right)\pi j},\frac{1}{5}e^{2\left(1/10\right)\pi j},\frac{1}{3}e^{2\left(1/4\right)\pi j}\right),\left(\left(d,f\right),\frac{1}{3}e^{2\left(1/20\right)\pi j},\frac{1}{5}e^{2\left(1/10\right)\pi j},\frac{1}{3}e^{2\left(1/4\right)\pi j}\right)\\ \left(\left(d,g\right),\frac{2}{7}e^{2\left(1/20\right)\pi j},\frac{1}{5}e^{2\left(1/10\right)\pi j},\frac{1}{3}e^{2\left(1/4\right)\pi j}\right),\left(\left(f,f\right),\frac{2}{5}e^{2\left(1/5\right)\pi j},\frac{2}{5}e^{2\left(3/10\right)\pi j},\frac{2}{10}e^{2\left(1/5\right)\pi j}\right)\\ \left(\left(g,f\right),\frac{2}{7}e^{2\left(1/10\right)\pi j},\frac{3}{10}e^{2\left(3/10\right)\pi j},\frac{1}{4}e^{2\left(1/5\right)\pi j}\right),\left(\left(g,g\right),\frac{2}{7}e^{2\left(1/10\right)\pi j},\frac{3}{10}e^{2\left(7/10\right)\pi j},\frac{1}{4}e^{2\left(1/6\right)\pi j}\right) \end{array}\right\}. \end{array}$$

**Definition 21 .**

A CPFR *R* is a complex picture strict order fuzzy relation (CP-strict order-FR) if *R* is

- CP-irreflexive-FR
- CP-transitive-FR

**Example 13 .**

The following relation *R* is a CP-strict order-FR on a CPFS *D* given in equation (20):

(30) $$\begin{array}{c} R=\left\{\begin{array}{c} \left(\left(d,f\right),\frac{1}{3}e^{2\left(1/20\right)\pi j},\frac{1}{5}e^{2\left(1/10\right)\pi j},\frac{1}{3}e^{2\left(1/4\right)\pi j}\right),\left(\left(d,g\right),\frac{2}{7}e^{2\left(1/20\right)\pi j},\frac{1}{5}e^{2\left(1/10\right)\pi j},\frac{1}{3}e^{2\left(1/4\right)\pi j}\right)\\ \left(\left(g,f\right),\frac{2}{7}e^{2\left(1/10\right)\pi j},\frac{3}{10}e^{2\left(3/10\right)\pi j},\frac{1}{4}e^{2\left(1/5\right)\pi j}\right) \end{array}\right\}. \end{array}$$

**Definition 22 .**

A CPFR *R* is a complex picture partial order fuzzy relation (CP-partial order-FR) if *R* is

- CP-reflexive-FR
- CP-antisymmetric-FR
- CP-transitive-FR

**Example 14 .**

RETRACTED

The following relation *R* is a CP-partial order-FR on a CPFS *D* given in equation (20):

(31) $$\begin{array}{c} R=\left\{\begin{array}{c} \left(\left(d,d\right),\frac{1}{3}e^{2\left(1/20\right)\pi j},\frac{1}{5}e^{2\left(1/10\right)\pi j},\frac{1}{3}e^{2\left(1/4\right)\pi j}\right),\left(\left(d,f\right),\frac{1}{3}e^{2\left(1/20\right)\pi j},\frac{1}{5}e^{2\left(1/10\right)\pi j},\frac{1}{3}e^{2\left(1/4\right)\pi j}\right)\\ \left(\left(f,f\right),\frac{2}{5}e^{2\left(1/5\right)\pi j},\frac{2}{5}e^{2\left(3/10\right)\pi j},\frac{2}{10}e^{2\left(1/5\right)\pi j}\right),\left(\left(g,d\right),\frac{2}{7}e^{2\left(1/20\right)\pi j},\frac{1}{5}e^{2\left(1/10\right)\pi j},\frac{1}{3}e^{2\left(1/4\right)\pi j}\right)\\ \left(\left(g,f\right),\frac{2}{7}e^{2\left(1/10\right)\pi j},\frac{3}{10}e^{2\left(3/10\right)\pi j},\frac{1}{4}e^{2\left(1/5\right)\pi j}\right),\left(\left(g,g\right),\frac{2}{7}e^{2\left(1/10\right)\pi j},\frac{3}{10}e^{2\left(7/10\right)\pi j},\frac{1}{4}e^{2\left(1/6\right)\pi j}\right) \end{array}\right\}. \end{array}$$

**Definition 23 .**

A CPFR *R* is a complex picture linear order fuzzy relation (CP-linear order-FR) if *R* is

- CP-reflexive-FR
- CP-antisymmetric-FR
- CP-transitive-FR
- CP-complete-FR

**Example 15 .**

The following relation *R* is a CP-antisymmetric-FR on a CPFS *D* given in equation (20):

(32) $$\begin{array}{c} R=\left\{\begin{array}{c} \left(\left(d,d\right),\frac{1}{3}e^{2\left(1/20\right)\pi j},\frac{1}{5}e^{2\left(1/10\right)\pi j},\frac{1}{3}e^{2\left(1/4\right)\pi j}\right),\left(\left(d,f\right),\frac{1}{3}e^{2\left(1/20\right)\pi j},\frac{1}{5}e^{2\left(1/10\right)\pi j},\frac{1}{3}e^{2\left(1/4\right)\pi j}\right)\\ \left(\left(d,g\right),\frac{2}{7}e^{2\left(1/20\right)\pi j},\frac{1}{5}e^{2\left(1/10\right)\pi j},\frac{1}{3}e^{2\left(1/4\right)\pi j}\right),\left(\left(f,f\right),\frac{2}{5}e^{2\left(1/5\right)\pi j},\frac{2}{5}e^{2\left(3/10\right)\pi j},\frac{2}{10}e^{2\left(1/5\right)\pi j}\right)\\ \left(\left(g,f\right),\frac{2}{7}e^{2\left(1/10\right)\pi j},\frac{3}{10}e^{2\left(3/10\right)\pi j},\frac{1}{4}e^{2\left(1/5\right)\pi j}\right),\left(\left(g,g\right),\frac{2}{7}e^{2\left(1/10\right)\pi j},\frac{3}{10}e^{2\left(7/10\right)\pi j},\frac{1}{4}e^{2\left(1/6\right)\pi j}\right) \end{array}\right\}. \end{array}$$

**Definition 24 .**

The composition of two CPFRs *R*_1_ and *R*_2_ is a complex picture composite fuzzy relation (CP-composite-FR) which is defined as follows:

(33) $$\begin{array}{c} \left(\left(d,f\right),\alpha_{M}\left(d,f\right)e^{2\rho_{M}\left(d,f\right)\pi j},\alpha_{A}\left(d,f\right)e^{2\rho_{A}\left(d,f\right)\pi j},\;\alpha_{N}\left(d,f\right)e^{2\rho_{N}\left(d,f\right)\pi j}\right)\in R_{1},\\ \left(\left(f,g\right),\alpha_{M}\left(f,g\right)e^{2\rho_{M}\left(f,g\right)\pi j},\alpha_{A}\left(f,g\right)e^{2\rho_{A}\left(f,g\right)\pi j},\;\alpha_{N}\left(f,g\right)e^{2\rho_{N}\left(f,g\right)\pi j}\right)\in R_{2}, \end{array}$$

and implies

(34) $$\begin{array}{c} \left(\left(d,g\right),\alpha_{M}\left(d,g\right)e^{2\rho_{M}\left(d,g\right)\pi j},\alpha_{A}\left(d,g\right)e^{2\rho_{A}\left(d,g\right)\pi j},\;\alpha_{N}\left(d,g\right)e^{2\rho_{N}\left(d,g\right)\pi j}\right)\in R_{1}\circ R_{2}. \end{array}$$

**Example 16 .**

RETRACTED

The following relation *R* is a CP-composite-FR between CPFRs *R*_1_ and *R*_2_:

(35) $$\begin{array}{c} R_{1}=\left\{\begin{array}{c} \left(\left(d,f\right),\frac{1}{3}e^{2\left(1/20\right)\pi j},\frac{1}{5}e^{2\left(1/10\right)\pi j},\frac{1}{3}e^{2\left(1/4\right)\pi j}\right),\left(\left(g,f\right),\frac{2}{7}e^{2\left(1/10\right)\pi j},\frac{3}{10}e^{2\left(3/10\right)\pi j},\frac{1}{4}e^{2\left(1/5\right)\pi j}\right) \end{array}\right\}\\ R_{2}=\left\{\begin{array}{c} \left(\left(d,d\right),\frac{1}{3}e^{2\left(1/20\right)\pi j},\frac{1}{5}e^{2\left(1/10\right)\pi j},\frac{1}{3}e^{2\left(1/4\right)\pi j}\right),\left(\left(d,f\right),\frac{1}{3}e^{2\left(1/20\right)\pi j},\frac{1}{5}e^{2\left(1/10\right)\pi j},\frac{1}{3}e^{2\left(1/4\right)\pi j}\right)\\ \left(\left(d,g\right),\frac{2}{7}e^{2\left(1/20\right)\pi j},\frac{1}{5}e^{2\left(1/10\right)\pi j},\frac{1}{3}e^{2\left(1/4\right)\pi j}\right),\left(\left(f,d\right),\frac{1}{3}e^{2\left(1/20\right)\pi j},\frac{1}{5}e^{2\left(1/10\right)\pi j},\frac{1}{3}e^{2\left(1/4\right)\pi j}\right)\\ \left(\left(f,f\right),\frac{2}{5}e^{2\left(1/5\right)\pi j},\frac{2}{5}e^{2\left(3/10\right)\pi j},\frac{2}{10}e^{2\left(1/5\right)\pi j}\right),\left(\left(g,f\right),\frac{2}{7}e^{2\left(1/10\right)\pi j},\frac{3}{10}e^{2\left(3/10\right)\pi j},\frac{1}{4}e^{2\left(1/5\right)\pi j}\right) \end{array}\right\},\\ R=R_{1}\circ R_{2}=\left\{\begin{array}{c} \left(\left(d,d\right),\frac{1}{3}e^{2\left(1/20\right)\pi j},\frac{1}{5}e^{2\left(1/10\right)\pi j},\frac{1}{3}e^{2\left(1/4\right)\pi j}\right),\left(\left(d,f\right),\frac{1}{3}e^{2\left(1/20\right)\pi j},\frac{1}{5}e^{2\left(1/10\right)\pi j},\frac{1}{3}e^{2\left(1/4\right)\pi j}\right)\\ \left(\left(g,d\right),\frac{2}{7}e^{2\left(1/20\right)\pi j},\frac{1}{5}e^{2\left(1/10\right)\pi j},\frac{1}{3}e^{2\left(1/4\right)\pi j}\right),\left(\left(g,f\right),\frac{2}{7}e^{2\left(1/10\right)\pi j},\frac{3}{10}e^{2\left(3/10\right)\pi j},\frac{1}{4}e^{2\left(1/5\right)\pi j}\right) \end{array}\right\}. \end{array}$$

**Definition 25 .**

RETRACTED

The equivalence class of *d* modulo *R* is defined as

(36) $$\begin{array}{c} R\left[d\right]=\left\{\begin{array}{c} \left(f,\alpha_{M}\left(f\right)e^{2\rho_{M}\left(f\right)\pi j},\alpha_{A}\left(f\right)e^{2\rho_{A}\left(f\right)\pi j},\;\alpha_{N}\left(f\right)e^{2\rho_{N}\left(f\right)\pi j}\right):\\ \left(\left(f,d\right),\alpha_{M}\left(f,d\right)e^{2\rho_{M}\left(f,d\right)\pi j},\alpha_{A}\left(f,d\right)e^{2\rho_{A}\left(f,d\right)\pi j},\;\alpha_{N}\left(f,d\right)e^{2\rho_{N}\left(f,d\right)\pi j}\right)\in R \end{array}\right\}, \end{array}$$

for (*d*, *α*_*M*_(*d*)*e*^2*ρ*_*M*_(*d*)*πj*^, *α*_*A*_(*d*)*e*^2*ρ*_*A*_(*d*)*πj*^,  *α*_*N*_(*d*)*e*^2*ρ*_*N*_(*d*)*πj*^) and a CP-equivalence-FR *R*.

**Example 17 .**

The following relation *R* is CP-equivalence-FR on a CPFS *D* given in equation (20):

(37) $$\begin{array}{c} R=\left\{\begin{array}{c} \left(\left(d,d\right),\frac{1}{3}e^{2\left(1/20\right)\pi j},\frac{1}{5}e^{2\left(1/10\right)\pi j},\frac{1}{3}e^{2\left(1/4\right)\pi j}\right),\left(\left(d,f\right),\frac{1}{3}e^{2\left(1/20\right)\pi j},\frac{1}{5}e^{2\left(1/10\right)\pi j},\frac{1}{3}e^{2\left(1/4\right)\pi j}\right)\\ \left(\left(f,d\right),\frac{1}{3}e^{2\left(1/20\right)\pi j},\frac{1}{5}e^{2\left(1/10\right)\pi j},\frac{1}{3}e^{2\left(1/4\right)\pi j}\right),\left(\left(f,f\right),\frac{2}{5}e^{2\left(1/5\right)\pi j},\frac{2}{5}e^{2\left(3/10\right)\pi j},\frac{2}{10}e^{2\left(1/5\right)\pi j}\right)\\ \left(\left(g,g\right),\frac{2}{7}e^{2\left(1/10\right)\pi j},\frac{3}{10}e^{2\left(7/10\right)\pi j},\frac{1}{4}e^{2\left(1/6\right)\pi j}\right) \end{array}\right\}. \end{array}$$

The equivalence classes of each element in *D* modulo *R* are

(38) $$\begin{array}{c} R\left[d\right]=\left\{\left(d,\frac{1}{3}e^{2\left(1/20\right)\pi j},\frac{1}{5}e^{2\left(1/10\right)\pi j},\frac{1}{3}e^{2\left(1/4\right)\pi j}\right),\left(f,\frac{2}{5}e^{2\left(1/5\right)\pi j},\frac{2}{5}e^{2\left(3/10\right)\pi j},\frac{1}{5}e^{2\left(1/5\right)\pi j}\right)\right\},\\ R\left[f\right]=\left\{\left(d,\frac{1}{3}e^{2\left(1/20\right)\pi j},\frac{1}{5}e^{2\left(1/10\right)\pi j},\frac{1}{3}e^{2\left(1/4\right)\pi j}\right),\left(f,\frac{2}{5}e^{2\left(1/5\right)\pi j},\frac{2}{5}e^{2\left(3/10\right)\pi j},\frac{1}{5}e^{2\left(1/5\right)\pi j}\right)\right\},\\ R\left[g\right]=\left\{\left(g,\frac{2}{7}e^{2\left(1/10\right)\pi j},\frac{3}{10}e^{2\left(7/10\right)\pi j},\frac{1}{4}e^{2\left(1/6\right)\pi j}\right)\right\}. \end{array}$$

## 4. Results

This section presents some results and properties of CP-symmetric-FRs, CP-transitive-FRs, CP-composite-FRs, and CP-equivalence-FRs.

RETRACTED

**Theorem 1 .**

A CPFR *R* is a CP-symmetric-FR on a CPFS *D*iff *R*=*R*^−1^.

**Proof**

Assume that *R* is a CP-symmetric-FR on a CPFS *D*, then

(39) $$\begin{array}{c} \left(\left(d,f\right),\alpha_{M}\left(d,f\right)e^{2\rho_{M}\left(d,f\right)\pi j},\alpha_{A}\left(d,f\right)e^{2\rho_{A}\left(d,f\right)\pi j},\;\alpha_{N}\left(d,f\right)e^{2\rho_{N}\left(d,f\right)\pi j}\right)\in R,\\ ⟺\left(\left(f,d\right),\alpha_{M}\left(f,d\right)e^{2\rho_{M}\left(f,d\right)\pi j},\alpha_{A}\left(f,d\right)e^{2\rho_{A}\left(f,d\right)\pi j},\;\alpha_{N}\left(f,d\right)e^{2\rho_{N}\left(f,d\right)\pi j}\right)\in R. \end{array}$$

However, ((*f*, *d*), *α*_*M*_(*f*, *d*)*e*^2*ρ*_*M*_(*f*, *d*)*πj*^, *α*_*A*_(*f*, *d*)*e*^2*ρ*_*A*_(*f*, *d*)*πj*^,  *α*_*N*_(*f*, *d*)*e*^2*ρ*_*N*_(*f*, *d*)*πj*^) ∈ *R*^−1^.

Therefore, *R*=*R*^−1^.

Conversely, assume that *R*=*R*^−1^, then

∀((*d*, *f*), *α*_*M*_(*d*, *f*)*e*^2*ρ*_*M*_(*d*, *f*)*πj*^, *α*_*A*_(*d*, *f*)*e*^2*ρ*_*A*_(*d*, *f*)*πj*^,  *α*_*N*_(*d*, *f*)*e*^2*ρ*_*N*_(*d*, *f*)*πj*^) ∈ *R*, and we have ((*f*, *d*), *α*_*M*_(*f*, *d*)*e*^2*ρ*_*M*_(*f*, *d*)*πj*^, *α*_*A*_(*f*, *d*)*e*^2*ρ*_*A*_(*f*, *d*)*πj*^,  *α*_*N*_(*f*, *d*)*e*^2*ρ*_*N*_(*f*, *d*)*πj*^) ∈ *R*^−1^ which implies that ((*f*, *d*), *α*_*M*_(*f*, *d*)*e*^2*ρ*_*M*_(*f*, *d*)*πj*^, *α*_*A*_(*f*, *d*)*e*^2*ρ*_*A*_(*f*, *d*)*πj*^,  *α*_*N*_(*f*, *d*)*e*^2*ρ*_*N*_(*f*, *d*)*πj*^) ∈ *R*.

So, *R* is a CP-symmetric-FR on *D*.

**Theorem 2 .**

. A CPFR *R* is a CP-transitive-FR on a CPFS *D*iff *R*∘*R*⊆*R*.

**Proof**

Assume that *R* is a CP-transitive-FR on a CPFS *D* and ((*d*, *g*), *α*_*M*_(*d*, *g*)*e*^2*ρ*_*M*_(*d*, *g*)*πj*^, *α*_*A*_(*d*, *g*)*e*^2*ρ*_*A*_(*d*, *g*)*πj*^,  *α*_*N*_(*d*, *g*)*e*^2*ρ*_*N*_(*d*, *g*)*πj*^) ∈ *R*∘*R*, then there exists an element *f* ∈ *Y* such that ((*d*, *f*), *α*_*M*_(*d*, *f*)*e*^2*ρ*_*M*_(*d*, *f*)*πj*^, *α*_*A*_(*d*, *f*)*e*^2*ρ*_*A*_(*d*, *f*)*πj*^,  *α*_*N*_(*d*, *f*)*e*^2*ρ*_*N*_(*d*, *f*)*πj*^) ∈ *R* and ((*f*, *g*), *α*_*M*_(*f*, *g*)*e*^2*ρ*_*M*_(*f*, *g*)*πj*^, *α*_*A*_(*f*, *g*)*e*^2*ρ*_*A*_(*f*, *g*)*πj*^,  *α*_*N*_(*f*, *g*)*e*^2*ρ*_*N*_(*f*, *g*)*πj*^) ∈ *R* which imply that

(40) $$\begin{array}{c} \left(\left(d,g\right),\alpha_{M}\left(d,g\right)e^{2\rho_{M}\left(d,g\right)\pi j},\alpha_{A}\left(d,g\right)e^{2\rho_{A}\left(d,g\right)\pi j},\;\alpha_{N}\left(d,g\right)e^{2\rho_{N}\left(d,g\right)\pi j}\right)\in R. \end{array}$$

Hence, *R*∘*R*⊆*R*.

Conversely, assume that *R*∘*R*⊆*R*, then the composition of CPFRs implies that

For ((*d*, *f*), *α*_*M*_(*d*, *f*)*e*^2*ρ*_*M*_(*d*, *f*)*πj*^, *α*_*A*_(*d*, *f*)*e*^2*ρ*_*A*_(*d*, *f*)*πj*^,  *α*_*N*_(*d*, *f*)*e*^2*ρ*_*N*_(*d*, *f*)*πj*^) ∈ *R* and ((*f*, *g*), *α*_*M*_(*f*, *g*)*e*^2*ρ*_*M*_(*f*, *g*)*πj*^, *α*_*A*_(*f*, *g*)*e*^2*ρ*_*A*_(*f*, *g*)*πj*^,  *α*_*N*_(*f*, *g*)*e*^2*ρ*_*N*_(*f*, *g*)*πj*^) ∈ *R*, we have

(41) $$\begin{array}{c} \left(\left(d,g\right),\alpha_{M}\left(d,g\right)e^{2\rho_{M}\left(d,g\right)\pi j},\alpha_{A}\left(d,g\right)e^{2\rho_{A}\left(d,g\right)\pi j},\;\alpha_{N}\left(d,g\right)e^{2\rho_{N}\left(d,g\right)\pi j}\right)\in R\circ R. \end{array}$$

Thus, the assumption implies the transitivity, i.e.,

(42) $$\begin{array}{c} R\circ R\subseteq R\Rightarrow \left(\left(d,g\right),\alpha_{M}\left(d,g\right)e^{2\rho_{M}\left(d,g\right)\pi j},\alpha_{A}\left(d,g\right)e^{2\rho_{A}\left(d,g\right)\pi j},\;\alpha_{N}\left(d,g\right)e^{2\rho_{N}\left(d,g\right)\pi j}\right)\in R. \end{array}$$

Hence, *R* is CP-transitive-FR.

RETRACTED

**Theorem 3 .**

If *R* is a CP-equivalence-FR on a CPFS *D*, then *R*∘*R*=*R*.

**Proof**

As *R* is a CP-equivalence-FR on a CPFS D, then

(43) $$\begin{array}{c} \left(\left(d,f\right),\alpha_{M}\left(d,f\right)e^{2\rho_{M}\left(d,f\right)\pi j},\alpha_{A}\left(d,f\right)e^{2\rho_{A}\left(d,f\right)\pi j},\;\alpha_{N}\left(d,f\right)e^{2\rho_{N}\left(d,f\right)\pi j}\right)\in R. \end{array}$$

The CP-symmetric-FR implies that

(44) $$\begin{array}{c} \left(\left(f,d\right),\alpha_{M}\left(f,d\right)e^{2\rho_{M}\left(f,d\right)\pi j},\alpha_{A}\left(f,d\right)e^{2\rho_{A}\left(f,d\right)\pi j},\;\alpha_{N}\left(f,d\right)e^{2\rho_{N}\left(f,d\right)\pi j}\right)\in R. \end{array}$$

The CP-transitive-FR implies that

(45) $$\begin{array}{c} \left(\left(d,d\right),\alpha_{M}\left(d,d\right)e^{2\rho_{M}\left(d,d\right)\pi j},\alpha_{A}\left(d,d\right)e^{2\rho_{A}\left(d,d\right)\pi j},\;\alpha_{N}\left(d,d\right)e^{2\rho_{N}\left(d,d\right)\pi j}\right)\in R. \end{array}$$

Also, the CP-composite-FR implies that

(46) $$\begin{array}{c} \left(\left(d,d\right),\alpha_{M}\left(d,d\right)e^{2\rho_{M}\left(d,d\right)\pi j},\alpha_{A}\left(d,d\right)e^{2\rho_{A}\left(d,d\right)\pi j},\;\alpha_{N}\left(d,d\right)e^{2\rho_{N}\left(d,d\right)\pi j}\right)\in R\circ R. \end{array}$$

Hence,

(47) $$\begin{array}{c} R\subseteq R\circ R. \end{array}$$

Conversely, assume that ((*d*, *g*), *α*_*M*_(*d*, *g*)*e*^2*ρ*_*M*_(*d*, *g*)*πj*^, *α*_*A*_(*d*, *g*)*e*^2*ρ*_*A*_(*d*, *g*)*πj*^,  *α*_*N*_(*d*, *g*)*e*^2*ρ*_*N*_(*d*, *g*)*πj*^) ∈ *R*∘*R*, then there exists an element *f* in *Y* such that

((*d*, *f*), *α*_*M*_(*d*, *f*)*e*^2*ρ*_*M*_(*d*, *f*)*πj*^, *α*_*A*_(*d*, *f*)*e*^2*ρ*_*A*_(*d*, *f*)*πj*^,  *α*_*N*_(*d*, *f*)*e*^2*ρ*_*N*_(*d*, *f*)*πj*^) ∈ *R* and ((*f*, *g*), *α*_*M*_(*f*, *g*)*e*^2*ρ*_*M*_(*f*, *g*)*πj*^, *α*_*A*_(*f*, *g*)*e*^2*ρ*_*A*_(*f*, *g*)*πj*^,  *α*_*N*_(*f*, *g*)*e*^2*ρ*_*N*_(*f*, *g*)*πj*^) ∈ *R*. *R* is a CP-equivalence-FR. Therefore, the CP-transitive-FR *R* implies that

(48) $$\begin{array}{c} \left(\left(d,g\right),\alpha_{M}\left(d,g\right)e^{2\rho_{M}\left(d,g\right)\pi j},\alpha_{A}\left(d,g\right)e^{2\rho_{A}\left(d,g\right)\pi j},\;\alpha_{N}\left(d,g\right)e^{2\rho_{N}\left(d,g\right)\pi j}\right)\in R. \end{array}$$

Hence,

(49) $$\begin{array}{c} R\circ R\subseteq R. \end{array}$$

Equations (47) and (49) prove assertion, i.e., *R*∘*R*=*R*.

RETRACTED

**Theorem 4 .**

If *R* is a CP-equivalence-FR on a CPFS *D*, then ((*d*, *f*), *α*_*M*_(*d*, *f*)*e*^2*ρ*_*M*_(*d*, *f*)*πj*^, *α*_*A*_(*d*, *f*)*e*^2*ρ*_*A*_(*d*, *f*)*πj*^,  *α*_*N*_(*d*, *f*)*e*^2*ρ*_*N*_(*d*, *f*)*πj*^) ∈ *R*iff *R*[*d*]=*R*[*f*].

**Proof**

*R* is a CP-equivalence-FR on a CPFS *D*. So, we can define the equivalence classes for *R*. Let *R*[*d*]=*R*[*f*], then for some *g* in *Y*,

(*g*, *α*_*M*_(*g*)*e*^2*ρ*_*M*_(*g*)*πj*^, *α*_*A*_(*g*)*e*^2*ρ*_*A*_(*g*)*πj*^,  *α*_*N*_(*g*)*e*^2*ρ*_*N*_(*g*)*πj*^) ∈ *R*[*d*] implies ((*g*, *d*), *α*_*M*_(*g*, *d*)*e*^2*ρ*_*M*_(*g*, *d*)*πj*^, *α*_*A*_(*g*, *d*)*e*^2*ρ*_*A*_(*g*, *d*)*πj*^,  *α*_*N*_(*g*, *d*)*e*^2*ρ*_*N*_(*g*, *d*)*πj*^) ∈ *R*.

By the definition of CP-symmetric-FR, we have

(50) $$\begin{array}{c} \left(\left(d,g\right),\alpha_{M}\left(d,g\right)e^{2\rho_{M}\left(d,g\right)\pi j},\alpha_{A}\left(d,g\right)e^{2\rho_{A}\left(d,g\right)\pi j},\;\alpha_{N}\left(d,g\right)e^{2\rho_{N}\left(d,g\right)\pi j}\right)\in R. \end{array}$$

Similarly,

(51) $$\begin{array}{c} \left(g,\alpha_{M}\left(g\right)e^{2\rho_{M}\left(g\right)\pi j},\alpha_{A}\left(g\right)e^{2\rho_{A}\left(g\right)\pi j},\;\alpha_{N}\left(g\right)e^{2\rho_{N}\left(g\right)\pi j}\right)\in R\left[f\right], \end{array}$$

which implies

(52) $$\begin{array}{c} \left(\left(g,f\right),\alpha_{M}\left(g,f\right)e^{2\rho_{M}\left(g,f\right)\pi j},\alpha_{A}\left(g,f\right)e^{2\rho_{A}\left(g,f\right)\pi j},\;\alpha_{N}\left(g,f\right)e^{2\rho_{N}\left(g,f\right)\pi j}\right)\in R. \end{array}$$

Using the definition of CP-transitive-FR on equations (50) and (52), we have

(53) $$\begin{array}{c} \left(\left(d,f\right),\alpha_{M}\left(d,f\right)e^{2\rho_{M}\left(d,f\right)\pi j},\alpha_{A}\left(d,f\right)e^{2\rho_{A}\left(d,f\right)\pi j},\;\alpha_{N}\left(d,f\right)e^{2\rho_{N}\left(d,f\right)\pi j}\right)\in R. \end{array}$$

Conversely, assume that

(54) $$\begin{array}{c} \left(\left(d,f\right),\alpha_{M}\left(d,f\right)e^{2\rho_{M}\left(d,f\right)\pi j},\alpha_{A}\left(d,f\right)e^{2\rho_{A}\left(d,f\right)\pi j},\;\alpha_{N}\left(d,f\right)e^{2\rho_{N}\left(d,f\right)\pi j}\right)\in R, \end{array}$$

(55) $$\begin{array}{c} \left(g,\alpha_{M}\left(g\right)e^{2\rho_{M}\left(g\right)\pi j},\alpha_{A}\left(g\right)e^{2\rho_{A}\left(g\right)\pi j},\;\alpha_{N}\left(g\right)e^{2\rho_{N}\left(g\right)\pi j}\right)\in R\left[d\right], \end{array}$$

which implies

(56) $$\begin{array}{c} \left(\left(g,d\right),\alpha_{M}\left(g,d\right)e^{2\rho_{M}\left(g,d\right)\pi j},\alpha_{A}\left(g,d\right)e^{2\rho_{A}\left(g,d\right)\pi j},\;\alpha_{N}\left(g,d\right)e^{2\rho_{N}\left(g,d\right)\pi j}\right)\in R. \end{array}$$

Using the definition of CP-transitive-FR on equations (54) and (56), we have

(57) $$\begin{array}{c} \left(\left(g,f\right),\alpha_{M}\left(g,f\right)e^{2\rho_{M}\left(g,f\right)\pi j},\alpha_{A}\left(g,f\right)e^{2\rho_{A}\left(g,f\right)\pi j},\;\alpha_{N}\left(g,f\right)e^{2\rho_{N}\left(g,f\right)\pi j}\right)\in R, \end{array}$$

which implies that (*g*, *α*_*M*_(*g*)*e*^2*ρ*_*M*_(*g*)*πj*^, *α*_*A*_(*g*)*e*^2*ρ*_*A*_(*g*)*πj*^,  *α*_*N*_(*g*)*e*^2*ρ*_*N*_(*g*)*πj*^) ∈ *R*[*f*].

RETRACTED

Hence,

(58) $$\begin{array}{c} R\left[d\right]\subseteq R\left[f\right]. \end{array}$$

Likewise, assume that

(59) $$\begin{array}{c} \left(\left(f,d\right),\alpha_{M}\left(f,d\right)e^{2\rho_{M}\left(f,d\right)\pi j},\alpha_{A}\left(f,d\right)e^{2\rho_{A}\left(f,d\right)\pi j},\;\alpha_{N}\left(f,d\right)e^{2\rho_{N}\left(f,d\right)\pi j}\right)\in R, \end{array}$$

(60) $$\begin{array}{c} \left(g,\alpha_{M}\left(g\right)e^{2\rho_{M}\left(g\right)\pi j},\alpha_{A}\left(g\right)e^{2\rho_{A}\left(g\right)\pi j},\;\alpha_{N}\left(g\right)e^{2\rho_{N}\left(g\right)\pi j}\right)\in R\left[f\right], \end{array}$$

which implies

(61) $$\begin{array}{c} \left(\left(g,f\right),\alpha_{M}\left(g,f\right)e^{2\rho_{M}\left(g,f\right)\pi j},\alpha_{A}\left(g,f\right)e^{2\rho_{A}\left(g,f\right)\pi j},\;\alpha_{N}\left(g,f\right)e^{2\rho_{N}\left(g,f\right)\pi j}\right)\in R. \end{array}$$

Using the definition of CP-transitive-FR on equations (59) and (61), we have

((*g*, *d*), *α*_*M*_(*g*, *d*)*e*^2*ρ*_*M*_(*g*, *d*)*πj*^, *α*_*A*_(*g*, *d*)*e*^2*ρ*_*A*_(*g*, *d*)*πj*^,  *α*_*N*_(*g*, *d*)*e*^2*ρ*_*N*_(*g*, *d*)*πj*^) ∈ *R*, which implies that (*g*, *α*_*M*_(*g*)*e*^2*ρ*_*M*_(*g*)*πj*^, *α*_*A*_(*g*)*e*^2*ρ*_*A*_(*g*)*πj*^,  *α*_*N*_(*g*)*e*^2*ρ*_*N*_(*g*)*πj*^) ∈ *R*[*d*].

Hence,

(62) $$\begin{array}{c} R\left[d\right]\subseteq R\left[f\right]. \end{array}$$

By equations (58) and (21), the assertion is proved, i.e., *R*[*d*]=*R*[*f*].

## 5. Applications

This section contains the applications of CPFSs, CPFRs, and their types.  Subsection 5.1 discusses an overview of the application problem and the algorithm of the application.  Subsection 5.2 lists and explains the securities that are considered for the problem. Further, Subsection 5.3 talks about the common threats that a network usually faces. In Subsection 5.4, the numerical analysis and solution to the problem are presented using the proposed methods.

RETRACTED

### 5.1. Network Security

Network security is an expansive word that covers a group of technologies, devices, techniques, and procedures. Network security can be defined in Layman's terms as a collection of rules and configurations that are designed to defend and safeguard the integrity, confidentiality, and accessibility of data and computer networks via software and hardware technologies. All industries, organizations, and enterprises require a degree of network security solutions to protect them from the expanding cyber threats in today's wild world.

In the following subsections, some common threats that are faced by networks, the network security techniques, and the relationships among them are discussed. The algorithm for the used method is portrayed through Figure 2. In words, Figure 2 can be described as follows:

  List the securities and the threats
  Make a set of securities and a set of threats that are to be studied
  Convert the two sets to CPFSs by carefully assigning each element the level of membership, level of abstinence, and level of nonmembership
  Find the Cartesian product between the two CPFSs
  Read and interpret the numerical results

### 5.2. Securities

Different methods of securing a network are discussed as follows. The level of membership, level of abstinence, and level of nonmembership are also assigned:

(1) *Network Access Control (NAC)*. NAC prevents the potential attackers from infiltrating the network. It is set at granular levels, e.g., granting administrators full access to the network and refusing access to particular private folders or stopping their personal devices from connecting to the network:
  (63) $$\begin{array}{c} \left(\text{NAC},\frac{1}{2}e^{\left(1/2\right)\pi j},\frac{1}{8}e^{\left(1/4\right)\pi j},\frac{1}{5}e^{\left(1/10\right)\pi j}\right). \end{array}$$
(2) *Antivirus (AV)*. Antivirus software keeps an organization protected from viruses, ransomware, worms, and Trojans:
  (64) $$\begin{array}{c} \left(\text{AV},\frac{3}{5}e^{\left(4/9\right)\pi j},\frac{1}{5}e^{\left(1/5\right)\pi j},\frac{2}{11}e^{\left(2/15\right)\pi j}\right). \end{array}$$
(3) *Firewall (FW)*. FW acts as a blockade between the trusted internal network and the untrusted external networks. The rules of blockade and authorization of traffic to a network are configured by administrators:
  (65) $$\begin{array}{c} \left(\text{FW},\frac{4}{7}e^{\left(2/3\right)\pi j},\frac{3}{14}e^{\left(1/6\right)\pi j},\frac{1}{7}e^{\left(1/10\right)\pi j}\right). \end{array}$$
(4) *Virtual Private Network (VPN)*. VPNs build a connection to the network from a different endpoint or location.
  (66) $$\begin{array}{c} \left(\text{VPN},\frac{1}{3}e^{\left(11/25\right)\pi j},\frac{1}{6}e^{\left(1/4\right)\pi j},\frac{3}{31}e^{\left(4/45\right)\pi j}\right). \end{array}$$

Table 2 contains the picture fuzzy information of above discussed securities.

RETRACTED

### 5.3. Threats

The most common network security threats one may encounter are explored as follows:

#### 5.3.1. Virus (**V**)

The most common network threats in cybersecurity for a daily Internet user are computer viruses. Generally, computer viruses are pieces of software and codes that are written to be spread from one computer to another. They disable security settings, send spam, corrupt, and steal data and information from a computer, and even they can delete everything on a hard drive. They enter through e-mail attachments or downloaded from specific websites to infect the computers on a network:

(67) $$\begin{array}{c} \left(V,\frac{3}{5}e^{\left(4/9\right)\pi j},\frac{1}{5}e^{\left(1/5\right)\pi j},\frac{2}{11}e^{\left(2/15\right)\pi j}\right). \end{array}$$

#### 5.3.2. Adware and Spyware (**A**&**S**)

Adware is any software which tracks data through browsing habits. Based on those habits, the advertisements and pop-ups are shown. The adware can slow down computer's processor and Internet connection speed. Adware downloaded without consent is considered malicious.

Spyware is similar to adware. It is secretly installed on a computer which contains key loggers for recording personal information such as e-mail addresses, passwords, and credit card information:

(68) $$\begin{array}{c} \left(A\&S,\frac{7}{11}e^{\left(1/2\right)\pi j},\frac{2}{11}e^{\left(1/4\right)\pi j},\frac{3}{22}e^{\left(1/6\right)\pi j}\right). \end{array}$$

#### 5.3.3. SQL Injection (SQL)

Many servers use SQL for storing website data. With the progression of technology, the network security threats have also advanced which lead the threat of SQL injection attacks.

SQL injection attacks exploit security vulnerabilities in the application's software to target data-bases. They use wicked code to achieve secretive data and change and even destroy that data. It is one of the most dangerous privacy issues for data confidentiality:

(69) $$\begin{array}{c} \left(\text{SQL},\frac{1}{2}e^{\left(2/3\right)\pi j},\frac{1}{4}e^{\left(1/5\right)\pi j},\frac{1}{5}e^{\left(1/10\right)\pi j}\right). \end{array}$$

#### 5.3.4. Trojan Horse (TH)

A Trojan horse or Trojan is a malicious bit of attacking code or software which is hidden behind a genuine program. It tricks people into running it willingly. They spread often by e-mail attachments and clicking on a false advertisement.

RETRACTED

It records passwords by logging keystrokes, hijack webcams, and steal sensitive data on a computer.

(70) $$\begin{array}{c} \left(\text{TH},\frac{1}{3}e^{\left(1/3\right)\pi j},\frac{1}{6}e^{\left(1/9\right)\pi j},\frac{1}{3}e^{\left(1/4\right)\pi j}\right). \end{array}$$

#### 5.3.5. Man-in-the-Middle (MITM)

Man-in-the-middle attacks are cybersecurity attacks that allow the attacker to eavesdrop on communication between two targets. It can listen to a private communication.

DNS spoofing, IP spoofing, ARP spoofing, HTTPS spoofing, Wi-Fi hacking, and SSL hijacking are some of the types of MITM attacks:

(71) $$\begin{array}{c} \left(\text{MITM},\frac{4}{13}e^{\left(3/7\right)\pi j},\frac{3}{7}e^{\left(3/7\right)\pi j},\frac{1}{3}e^{\left(1/7\right)\pi j}\right). \end{array}$$

Table 3 contains the picture fuzzy information of above discussed threats.

### 5.4. Calculations

Now that, the effectiveness and ineffectiveness of each network security and threat are analyzed, and we carry out the following mathematics.

Since we have the following two CPFSs, *S* and *T* that represent the sets of securities and threats, respectively, are as follows:

(72) $$\begin{array}{c} S=\left\{\begin{array}{c} \left(\text{NAC},\frac{1}{2}e^{\left(1/2\right)\pi j},\frac{1}{8}e^{\left(1/4\right)\pi j},\frac{1}{5}e^{\left(1/10\right)\pi j}\right),\left(\text{AV},\frac{3}{5}e^{\left(4/9\right)\pi j},\frac{1}{5}e^{\left(1/5\right)\pi j},\frac{2}{11}e^{\left(2/15\right)\pi j}\right)\\ \left(\text{FW},\frac{4}{7}e^{\left(2/3\right)\pi j},\frac{3}{14}e^{\left(\frac{1}{6}\right)\pi j},\frac{1}{7}e^{\left(1/10\right)\pi j}\right),\left(\text{VPN},\frac{1}{3}e^{\left(11/25\right)\pi j},\frac{1}{6}e^{\left(1/4\right)\pi j},\frac{3}{31}e^{\left(4/45\right)\pi j}\right) \end{array}\right\}.\\ T=\left\{\begin{array}{c} \left(V,\frac{3}{5}e^{\left(4/9\right)\pi j},\frac{1}{5}e^{\left(1/5\right)\pi j},\frac{2}{11}e^{\left(2/15\right)\pi j}\right),\left(A\&S,\frac{7}{11}e^{\left(1/2\right)\pi j},\frac{2}{11}e^{\left(1/4\right)\pi j},\frac{3}{22}e^{\left(1/6\right)\pi j}\right)\\ \left(\text{SQL},\frac{1}{2}e^{\left(2/3\right)\pi j},\frac{1}{4}e^{\left(1/5\right)\pi j},\frac{1}{5}e^{\left(1/10\right)\pi j}\right),\left(\text{TH},\frac{1}{3}e^{\left(1/3\right)\pi j},\frac{1}{6}e^{\left(1/9\right)\pi j},\frac{1}{3}e^{\left(1/4\right)\pi j}\right)\\ \left(\text{MITM},\frac{4}{13}e^{\left(3/7\right)\pi j},\frac{3}{7}e^{\left(3/7\right)\pi j},\frac{1}{3}e^{\left(1/7\right)\pi j}\right) \end{array}\right\}. \end{array}$$

The conception of Cartesian product is used to find out the ability of certain securities against specific threat. Thus, finding the Cartesian product between the CPFSs *S* and *T* is deliberated by Table 4.

RETRACTED

Each pair of elements in the Cartesian product *S* × *T* describes the association between that pair, i.e., the influences and impacts of a security on a threat. The levels of membership tell the efficacy of a network security to grab a specific threat with respect to some time. The levels of abstinence indicate the no effects or neutral effect of a security against a certain threat. The levels of nonmembership designate the inefficiency or ineptness of a security against a certain threat. For example, the ordered pair ((AV, *V*), (3/5)*e*^(4/9)*πj*^, (1/5)*e*^(1/5)*πj*^, (2/11)*e*^(2/15)*πj*^) emphasizes that the antivirus software can positively tackle the threats and risks to the network by viruses. Further, the numbers explain that the levels of uselessness and inefficiency are low, i.e., the levels of abstinence and nonmembership, respectively. More precisely, the complex picture fuzzy values are translated as the level of security that antivirus software provides against the vulnerabilities of a virus is 60% with respect to (4/9) time units, the level of neutral effects is 20% with respect to 1/5 time units, and the chances of risks via viruses evading the antivirus software are 18% with respect to 2/15 time units. In case of the securities, the longer durations of time in the level of membership is thought to be better, while the smaller time frame in the levels of nonmembership is better. Obviously, the levels of abstinence describe the neutral effects.

## 6. Comparative Analysis

In this section, the reliability of the proposed structures of CPFRs is verified by carrying out the comparative study among the proposed and preexisting structures such as FRs, CFRs, IFRs, CIFRs, and PFRs.

### 6.1. Comparison with FRs, IFRs, and PFRs

The structures of FR, IFR, and PFR have one similarity, that is, the real-valued level of memberships, level of abstinence, and level of nonmemberships. Therefore, they are limited to only one-dimensional problems. These structures cannot model periodicity and problems with multivariable.

FRs only discuss the level of membership. IFRs discuss the level of membership and level of nonmembership. So, these structures are completely swept out of the competition.

On the other hand, PFRs discuss all the three levels, i.e., level of membership, level of abstinence, and level of nonmembership. A detailed comparison is given as follows.

Let us consider the problem deliberated in Section 5.4 by using PFRs. Think of the two PFSs *S* and *T* representing the set of securities and the set of threats, respectively:

(73) $$\begin{array}{c} S=\left\{\begin{array}{c} \left(\text{NAC},\frac{1}{2},\frac{1}{8},\frac{1}{5}\right),\left(\text{AV},\frac{3}{5},\frac{1}{5},\frac{2}{11}\right),\left(\text{FW},\frac{4}{7},\frac{3}{14},\frac{1}{7}\right),\left(\text{VPN},\frac{1}{3},\frac{1}{6},\frac{3}{31}\right) \end{array}\right\},\\ T=\left\{\begin{array}{c} \left(V,\frac{3}{5},\frac{1}{5},\frac{2}{11}\right),\left(A\&S,\frac{7}{11},\frac{2}{11},\frac{3}{22}\right),\left(\text{SQL},\frac{1}{2},\frac{1}{4},\frac{1}{5}\right),\left(\text{TH},\frac{1}{3},\frac{1}{6},\frac{1}{3}\right),\left(\text{MITM},\frac{4}{13},\frac{3}{7},\frac{1}{3}\right) \end{array}\right\}. \end{array}$$

Table 5 contains the details of abbreviations used in the above sets.

RETRACTED

The PFR *R* between *S* and *T* is given in Table 6.

It is clear from the above PFR *R* that it gives the real-valued information of level of membership, level of abstinence, and level of nonmembership. So, it does not indicate the time frame for the relation.

Hence, these structures have certain limitations, and thus they give limited information.

### 6.2. Comparison with CFRs and CIFRs

The structures of CFR and CIFR consist of complex valued functions.

The CFRs only discuss the level of membership. Therefore, they cannot provide sufficient solution to the problem in application.

The CIFR talks about the level of membership and level of nonmembership. Thus, CIFRs are used to solve the problem in Section 5.4.

Let us consider the problem deliberated in Section 5.4 by using CIFRs. Think of the two CIFSs *S* and *T* representing the set of securities and the set of threats, respectively:

(74) $$\begin{array}{c} S=\left\{\begin{array}{c} \left(\text{NAC},\frac{1}{2}e^{\left(1/2\right)\pi j},\frac{1}{5}e^{\left(1/10\right)\pi j}\right),\left(\text{AV},\frac{3}{5}e^{\left(4/9\right)\pi j},\frac{2}{11}e^{\left(2/15\right)\pi j}\right)\\ \left(\text{FW},\frac{4}{7}e^{\left(2/3\right)\pi j},\frac{1}{7}e^{\left(1/10\right)\pi j}\right),\left(\text{VPN},\frac{1}{3}e^{\left(11/25\right)\pi j},\frac{3}{31}e^{\left(4/45\right)\pi j}\right) \end{array}\right\},\\ T=\left\{\begin{array}{c} \left(V,\frac{3}{5}e^{\left(4/9\right)\pi j},\frac{2}{11}e^{\left(2/15\right)\pi j}\right),\left(A\&S,\frac{7}{11}e^{\left(1/2\right)\pi j},\frac{3}{22}e^{\left(1/6\right)\pi j}\right),\left(\text{SQL},\frac{1}{2}e^{\left(2/3\right)\pi j},\frac{1}{5}e^{\left(1/10\right)\pi j}\right)\\ \left(\text{TH},\frac{1}{3}e^{\left(1/3\right)\pi j},\frac{1}{3}e^{\left(1/4\right)\pi j}\right),\left(\text{MITM},\frac{4}{13}e^{\left(3/7\right)\pi j},\frac{1}{3}e^{\left(1/7\right)\pi j}\right) \end{array}\right\}. \end{array}$$

The details of abbreviations used in the above sets are described in Table 5.

RETRACTED

The CIFR *R* between *S* and *T* is given in Table 7.

It is clear from Table 7 that the abovementioned structures cannot model the problem as efficiently as CPFR. However, a CPFR provides relatively more detailed informations about the relationship. Hence, these structures have certain limitations, and they give limited information.

Table 8 gives the summary of characteristics of ten different structures in fuzzy set theory. From Table 8, the supremacy of the structure of CPFRs is proved. It ticks all the four characteristics, while the rest of the competitors have limitations in their structures.

## 7. Conclusion

This article introduced the novel concepts of complex picture fuzzy relations (CPFRs) using the idea of Cartesian products between two complex picture fuzzy sets (CPFSs). Moreover, the types of CPFRs such as CP-equivalence-FR, CP-partial order-FR, CP-total order-FR, and CP-composite-FR were also studied with the help of definitions, suitable examples, properties, and results. Furthermore, the ground-breaking modeling techniques, based on the proposed picture fuzzy information, were introduced. These modeling methods were then used to model the problems of network and communication securities. The application problem was modeled and solved to achieve the required results, i.e., the level of effectiveness, ineffectiveness, and no effects of the network security methods against the threats that are faced by the network and communication systems. Finally, a comparative study had been carried out that verified the preeminence of the proposed methods over the existing methods. In future, these innovative concepts can be further extended to other generalizations of fuzzy set theory and fuzzy logic which will produce robust modeling techniques.

## Figures and Tables

**Figure 1:** Steps involved in the proposed modeling technique.

**Figure 2:** Flowchart for the process being followed.

**Table 1:** Organization of the article.

Section	Description
1	Introduction and literature review
2	Preliminaries; in this section, predefined concepts are reviewed to provide a base for the proposed work
3	This section defines the novel concepts of complex picture fuzzy relations and their types with examples
4	Some results and properties of the proposed notions are discussed
5	An application of communication and network securities is presented
6	The comparison among the preexisting and the proposed structures is carried out. The application problem is solved by different methods and techniques which fail to produce the required results
7	Conclusion to the article

RETRACTED

**Table 2:** Picture fuzzy information of securities.

Security	Abbreviation	Membership	Abstinence	Nonmembership
Network access control	NAC	(1/2)*e*^(1/2)*πj*^	(1/8)*e*^(1/4)*πj*^	(1/5)*e*^(1/10)*πj*^
Antivirus	AV	(3/5)*e*^(4/9)*πj*^	(1/5)*e*^(1/5)*πj*^	(2/11)*e*^(2/15)*πj*^
Firewall	FW	(4/7)*e*^(2/3)*πj*^	(3/14)*e*^(1/6)*πj*^	(1/7)*e*^(1/10)*πj*^
Virtual private network	VPN	(1/3)*e*^(11/25)*πj*^	(1/6)*e*^(1/4)*πj*^	(3/31)*e*^(4/45)*πj*^

**Table 3:** Picture fuzzy information of threats.

Security	Abbreviation	Membership	Abstinence	Nonmembership
Virus	*V*	(3/5)*e*^(4/9)*πj*^	(1/5)*e*^(1/5)*πj*^	(2/11)*e*^(2/15)*πj*^
Adware and spyware	*A*&*S*	(7/11)*e*^(1/2)*πj*^	(2/11)*e*^(1/4)*πj*^	(3/22)*e*^(1/6)*πj*^
SQL injection	SQL	(1/2)*e*^(2/3)*πj*^	(1/4)*e*^(1/5)*πj*^	(1/5)*e*^(1/10)*πj*^
Trojan horse	TH	(1/3)*e*^(1/3)*πj*^	(1/6)*e*^(1/9)*πj*^	(1/3)*e*^(1/4)*πj*^
Man-in-the-middle	MITM	(4/13)*e*^(3/7)*πj*^	(3/7)*e*^(3/7)*πj*^	(1/3)*e*^(1/7)*πj*^

**Table 4:** Cartesian product between *S* and *T*.

Relation elements	Membership	Abstinence	Nonmembership
(NAC, *V*)	(1/2)*e*^(4/9)*πj*^	(1/8)*e*^(1/5)*πj*^	(1/5)*e*^(2/15)*πj*^
(NAC, *A*&*S*)	(1/2)*e*^(1/2)*πj*^	(1/8)*e*^(1/4)*πj*^	(1/5)*e*^(1/6)*πj*^
(NAC, SQL)	(1/2)*e*^(1/2)*πj*^	(1/8)*e*^(1/5)*πj*^	(1/5)*e*^(1/10)*πj*^
(NAC, TH)	(1/3)*e*^(1/3)*πj*^	(1/8)*e*^(1/9)*πj*^	(1/3)*e*^(1/4)*πj*^
(NAC, MITM)	(4/13)*e*^(3/7)*πj*^	(1/8)*e*^(1/4)*πj*^	(1/3)*e*^(1/7)*πj*^
(AV, *V*)	(3/5)*e*^(4/9)*πj*^	(1/5)*e*^(1/5)*πj*^	(2/11)*e*^(2/15)*πj*^
(AV, *A*&*S*)	(3/5)*e*^(4/9)*πj*^	(2/11)*e*^(1/5)*πj*^	(2/11)*e*^(1/6)*πj*^
(AV, SQL)	(1/2)*e*^(4/9)*πj*^	(1/5)*e*^(1/5)*πj*^	(1/5)*e*^(2/15)*πj*^
(AV, TH)	(1/3)*e*^(1/3)*πj*^	(1/6)*e*^(1/9)*πj*^	(1/3)*e*^(1/4)*πj*^
(AV, MITM)	(4/13)*e*^(3/7)*πj*^	(1/5)*e*^(1/5)*πj*^	(1/3)*e*^(1/7)*πj*^
(FW, *V*)	(4/7)*e*^(4/9)*πj*^	(1/5)*e*^(1/6)*πj*^	(2/11)*e*^(2/15)*πj*^
(FW, *A*&*S*)	(4/7)*e*^(1/2)*πj*^	(2/11)*e*^(1/6)*πj*^	(1/7)*e*^(1/6)*πj*^
(FW, SQL)	(1/2)*e*^(2/3)*πj*^	(3/14)*e*^(1/6)*πj*^	(1/5)*e*^(1/10)*πj*^
(FW, TH)	(1/3)*e*^(1/3)*πj*^	(1/6)*e*^(1/9)*πj*^	(1/3)*e*^(1/4)*πj*^
(FW, MITM)	(4/13)*e*^(3/7)*πj*^	(3/14)*e*^(1/6)*πj*^	(1/3)*e*^(1/7)*πj*^
(VPN, *V*)	(1/3)*e*^(11/25)*πj*^	(1/6)*e*^(1/5)*πj*^	(2/11)*e*^(2/15)*πj*^
(VPN, *A*&*S*)	(1/3)*e*^(11/25)*πj*^	(1/6)*e*^(1/4)*πj*^	(3/22)*e*^(1/6)*πj*^
(VPN, SQL)	(1/3)*e*^(11/25)*πj*^	(1/6)*e*^(1/5)*πj*^	(1/5)*e*^(1/10)*πj*^
(VPN, TH)	(1/3)*e*^(1/3)*πj*^	(1/6)*e*^(1/9)*πj*^	(1/3)*e*^(1/4)*πj*^
(VPN, MITM)	(4/13)*e*^(3/7)*πj*^	(1/6)*e*^(1/4)*πj*^	(1/3)*e*^(1/7)*πj*^

**Table 5:** Abbreviations.

Abbreviations	Full names
NAC	Network access control
AV	Antivirus
FW	Firewall
VPN	Virtual private network
*V*	Virus
*A*&*S*	Adware and spyware
SQL	SQL injection
TH	Trojan horse
MITM	Man-in-the-middle

RETRACTED

**Table 6:** The PFR *R* between *S* and *T*.

Relation elements	Membership	Abstinence	Nonmembership
(NAC, *V*)	1/2	1/8	1/5
(NAC, *A*&*S*)	1/2	1/8	1/5
(NAC, SQL)	1/2	1/8	1/5
(NAC, TH)	1/3	1/8	1/3
(NAC, MITM)	4/13	1/8	1/3
(AV, *V*)	3/5	1/5	2/11
(AV, *A*&*S*)	3/5	2/11	2/11
(AV, SQL)	1/2	1/5	1/5
(AV, TH)	1/3	1/6	1/3
(AV, MITM)	4/13	1/5	1/3
(FW, *V*)	4/7	1/5	2/11
(FW, *A*&*S*)	4/7	2/11	1/7
(FW, SQL)	1/2	3/14	1/5
(FW, TH)	1/3	1/6	1/3
(FW, MITM)	4/13	3/14	1/3
(VPN, *V*)	1/3	1/6	2/11
(VPN, *A*&*S*)	1/3	1/6	3/22
(VPN, SQL)	1/3	1/6	1/5
(VPN, TH)	1/3	1/6	1/3
(VPN, MITM)	4/13	1/6	1/3

**Table 7:** The CIFR *R* between *S* and *T*.

Relation elements	Membership	Nonmembership
(NAC, *V*)	(1/2)*e*^(4/9)*πj*^	(1/5)*e*^(2/15)*πj*^
(NAC, *A*&*S*)	(1/2)*e*^(1/2)*πj*^	(1/5)*e*^(1/6)*πj*^
(NAC, SQL)	(1/2)*e*^(1/2)*πj*^	(1/5)*e*^(1/10)*πj*^
(NAC, TH)	(1/3)*e*^(1/3)*πj*^	(1/3)*e*^(1/4)*πj*^
(NAC, MITM)	(4/13)*e*^(3/7)*πj*^	(1/3)*e*^(1/7)*πj*^
(AV, *V*)	(3/5)*e*^(4/9)*πj*^	(2/11)*e*^(2/15)*πj*^
(AV, *A*&*S*)	(3/5)*e*^(4/9)*πj*^	(2/11)*e*^(1/6)*πj*^
(AV, SQL)	(1/2)*e*^(4/9)*πj*^	(1/5)*e*^(2/15)*πj*^
(AV, TH)	(1/3)*e*^(1/3)*πj*^	(1/3)*e*^(1/4)*πj*^
(AV, MITM)	(4/13)*e*^(3/7)*πj*^	(1/3)*e*^(1/7)*πj*^
(FW, *V*)	(4/7)*e*^(4/9)*πj*^	(2/11)*e*^(2/15)*πj*^
(FW, *A*&*S*)	(4/7)*e*^(1/2)*πj*^	(1/7)*e*^(1/6)*πj*^
(FW, SQL)	(1/2)*e*^(2/3)*πj*^	(1/5)*e*^(1/10)*πj*^
(FW, TH)	(1/3)*e*^(1/3)*πj*^	(1/3)*e*^(1/4)*πj*^
(FW, MITM)	(4/13)*e*^(3/7)*πj*^	(1/3)*e*^(1/7)*πj*^
(VPN, *V*)	(1/3)*e*^(11/25)*πj*^	(2/11)*e*^(2/15)*πj*^
(VPN, *A*&*S*)	(1/3)*e*^(11/25)*πj*^	(3/22)*e*^(1/6)*πj*^
(VPN, SQL)	(1/3)*e*^(11/25)*πj*^	(1/5)*e*^(1/10)*πj*^
(VPN, TH)	(1/3)*e*^(1/3)*πj*^	(1/3)*e*^(1/4)*πj*^
(VPN, MITM)	(4/13)*e*^(3/7)*πj*^	(1/3)*e*^(1/7)*πj*^

**Table 8:** Comparison on the basis of structural properties.

Structure	Membership	Abstinence	Nonmembership	Multidimensional	Remarks
FR	✓	✗	✗	✗	Only discusses membership with single variable
CFR	✓	✗	✗	✓	Only discusses membership with multivariable
IFR	✓	✗	✓	✗	Only discusses membership and nonmembership with single variable
CIFR	✓	✗	✓	✓	Only discusses membership and nonmembership with multivariable
PFR	✓	✓	✓	✗	Discusses membership, abstinence, and nonmembership but with single variable
CPFR	✓	✓	✓	✓	Discusses membership, abstinence, and nonmembership with multivariable

## Data Availability

Data sharing is not applied to this article as no data set was generated or analyzed during the current study.
